The article "Effects of the Alpha, Beta, and Gamma Binaural Beat Brain Stimulation and Short-Term Training on Simultaneously Assessed Visuospatial and Verbal Working Memories, Signal Detection Measures, Response Times, and Intrasubject Response Time Variabilities: A Within-Subject Randomized Placebo-Controlled Clinical Trial" was published in 2022. Journal: Biomed Res Int.

# Effects of the Alpha, Beta, and Gamma Binaural Beat Brain Stimulation and Short-Term Training on Simultaneously Assessed Visuospatial and Verbal Working Memories, Signal Detection Measures, Response Times, and Intrasubject Response Time Variabilities: A Within-Subject Randomized Placebo-Controlled Clinical Trial

**DOI:** 10.1155/2022/8588272

**Published:** 2022-04-22

**Authors:** Vahid Rakhshan, Peyman Hassani-Abharian, Mohammadtaghi Joghataei, Mohammad Nasehi, Reza Khosrowabadi

**Affiliations:** ^1^Department of Cognitive Neuroscience, Institute for Cognitive Science Studies, Tehran, Iran; ^2^Department of Cognitive Rehabilitation, Institute for Cognitive Science Studies, Tehran, Iran; ^3^Cellular and Molecular Research Center, Department of Neuroscience, Faculty of Advance Technology in Medicine, Iran University of Medical Sciences, Tehran, Iran; ^4^Cognitive and Neuroscience Research Center (CNRC), Tehran Medical Sciences, Islamic Azad University, Tehran, Iran; ^5^Institute for Cognitive and Brain Sciences, Shahid Beheshti University, Tehran, Iran

## Abstract

**Introduction:**

Binaural beats (BBs) are phantom sound illusions perceived when two sounds of slightly different frequencies are separately transmitted to the ears. It is suggested that some BB frequencies might entrain the brain and enhance certain cognitive functions such as working memory or attention. Nevertheless, studies in this regard are very scarce, quite controversial, and merely covering a very small portion of this vast field of research (e.g., testing only a few BB frequencies), not to mention adopting some limited methodologies (e.g., no assessment of the loudness of the BB sound, adopting only between-subject analyses, and testing only one perceptual modality). Hence, we aimed to assess the potential effects of alpha, beta, and gamma BBs on cognitive-behavioral parameters of working memory and attention examined simultaneously in two different modalities (visuospatial and auditory-verbal).

**Methods:**

This within-subject five-arm randomized placebo-controlled clinical trial included 155 trials in 31 healthy right-handed subjects (17 women, 14 men, 30.84 ± 6.16 years old). Each subject listened to 8-minute sessions of 10 Hz, 16 Hz, and 40 Hz binaural beats versus 240 Hz pure tone and silence (in random orders). In each 8-minute block, they played a dual 2-back task with feedback enabled. Their cognitive-behavioral parameters (working memory capacities, signal detection measures (hit rate, false alarm rate, sensitivity, and response bias), and reaction speed measures (response time and intrasubject response time variability)) were calculated. The effects of the sound interventions and short-term training on these working memory and attention measures were assessed statistically using mixed-model linear regressions, repeated-measures ANOVAs and ANCOVAs, Bonferroni *post hoc* tests, and one-sample *t*-tests (*α* = 0.05).

**Results:**

The following are some major statistically significant findings (*P* ≤ 0.05): In the visuospatial modality, the 10 Hz BB reduced the response time and intrasubject response time variability and reduced the extent of decline over time in the case of visuospatial working memory, sensitivity, and hit rate. In the auditory-verbal modality, the 10 Hz intervention reduced the hit rate, false alarm rate, and sensitivity. The 10 Hz intervention also caused the lowest intermodality discrepancies in hit rates and false alarm rates, the highest response time discrepancies, and negative discrepancies in working memories and sensitivities (indicating the superiority of the visuospatial modality). The response biases tended to be liberal-to-neutral in the verbal modality and rather conservative in the visuospatial modality. Reactions were faster in the visuospatial modality than the auditory-verbal one, while the intrasubject variability of reaction times was smaller in the auditory-verbal modality. Short-term training can increase the hit rate, working memory, and sensitivity and can decrease the false alarm rate and response time. Aging and reduced sound intervention volume may slow down responses and increase the intrasubject variability of response time. Faster reactions might be correlated with greater hit rates, working memories, and sensitivities and also with lower false alarm rates.

**Conclusions:**

The 8-minute alpha-band binaural beat entrainment may have a few, slight enhancing effects within the visuospatial modality, but not in both modalities combined. Short-term training can improve working memory and some cognitive parameters of attention. Some BB interventions can affect the intermodality discrepancies. There may be differences between the two modalities in terms of the response speeds and intrasubject response time variabilities. Aging can slow down the response, while increasing the volume of audio interventions may accelerate it.

## 1. Introduction

Working memory is one of the most fundamental and recognized cognitive functions and is known as the foundation of thinking and learning [1–3]. It is the system controlling the online organization and processing of information to temporarily hold, process, and operate information for effective comprehension, reasoning, decision-making, problem-solving, goal-directed behavior, language, solving arithmetical problems, understanding geometric analogies, etc. [3–9], and it is associated with many indices such as fluid intelligence, academic performance, and effective behavior [3]. Therefore, strengthening working memory (WM) can enhance the quality of numerous cognitive and behavioral outcomes.

Rhythm, music, and audio stimuli, in general, are used by humans to improve cognitive performances and enhance moods while studying or in social gatherings [10–13]. A new type of audio stimulus is binaural beats. Binaural beats are a form of auditory illusion; they form when the brain attempts to localize the source of a sound while two pure tones slightly different in frequency are relayed independently to each ear. In this case, a third phantom binaural beat with a frequency equal to the discrepancy between the two independent sounds is generated in the Inferior Colliculus [14], which projects it to the primary auditory cortex [15–18]. It is claimed that they may influence different cognitive functions and mood states, like memory, attention, vigilance, and creativity [16, 19], perhaps through alterations in the functioning of different brain networks as a result of synchronized hemispheric oscillations and brainwave entrainment [4, 16, 20–24]. Therefore, binaural beats are being introduced as a new potential cognitive booster that might also have various influences such as changing the mood [10], altering the states of consciousness [25], or entraining the whole brain [26, 27] (although recent studies failed to find mood-altering effects [28]). The noninvasive nature of these stimuli, their inexpensiveness, their ease of administration, and their potential ability to modulate cognition without previous training make binaural beats an intriguing candidate for use by both impaired and healthy individuals [10].

Therefore, binaural beats (BBs) might be used to enhance the working memory capacity. However, studies in this regard are few, quite controversial, and limited by methodologies and methodological differences (e.g., a study had enrolled only 4 subjects; all studies had merely between-subject analyses; only a few BB frequencies were ever researched, and the effects of many other binaural beat frequencies remain to be examined; each study has used a different measure of working memory; the duration of exposure to binaural beats differed among studies; and in most studies, the effect of binaural beats had been examined after the exposure to them and not during their exposure). Moreover, no study to date has assessed both visuospatial and auditory-verbal working memories simultaneously. Finally, none so far has assessed the effect of the intervention sound volume: previous studies which had reported the level of sound volume had either fixed the sound volume or adjusted it to the maximum loudness that could be comfortably heard by the subject. The constant sound volume in the former case could be too loud and discomforting for some subjects while too quiet for some other subjects, being suboptimum and interfering with results in both conditions, whereas, in the latter case, the effect of the customized sound volume itself should have been accounted for statistically; however, this had not happened.

There are merely 6 controversial studies on the effects of a few binaural beat frequencies on heterogeneous measures of working memory: Beauchene et al. [4, 16] assessed the effects of 5-minute sessions of binaural beat stimulation separately on verbal and visuospatial working memories. They concluded in two separate studies that 5-minute induction of binaural beats at merely 15 Hz (but not at 5 Hz or 10 Hz) could increase both verbal work memory and delta accuracy in a visuospatial working memory task (delta being the difference between accuracies estimated in the last and first thirds of the 5-minute session), in comparison with classical music, pure tone, and silence [4, 16]. It should be noted that their raw accuracy measures did not show any significance, and their significant findings were on measures such as delta accuracy and ranked accuracy. Moreover, their statistically significant findings in both articles might have been erroneous, as they seemed to have used between-subject statistical analyses for a within-subject (repeated-measures) design, besides other errors. Unlike their results, Ortiz et al. [29] (who evaluated the effects of binaural beats before and during the task (for a total of 15 minutes a day, for 5 days) on verbal working memory) observed an improved function under theta frequencies compared to beta binaural beats or white noise. As another addition to the dispute, Kraus and Porubanova [30] assessed the influence of 12-minute sessions of binaural beats at 9.55 Hz merged with the sound of the sea compared to a 12-minute control sound of the sea alone while examining the working memory performance using the Automated Operation Span Task (AOSPAN). The binaural beat intervention improved the working memory of participants. In another study comparing the effects of the exposure to 30 minutes of beta versus theta frequencies of binaural beats on the working memory, Lane et al. [31] had their participants run vigilance tasks. Their findings indicated that theta beats might increase fatigue, confusion, and difficulty concentrating, while beta beats might decrease false alarms, confusion, and fatigue while improving target detection [31]. Wahbeh et al. [23] assessed the effects of exposure to 30 minutes of theta binaural beats while testing the verbal memory of 4 subjects using the Rey Auditory Verbal Learning Test (RAVLT). They observed that pink noise exposure in the control group had a better result compared to binaural beats.

This randomized clinical trial was conducted because of the following reasons as well as shortcomings in the literature: (1) The improvement of working memory and other cognitive-behavioral functions using noninvasive and inexpensive methods such as the binaural beat stimulation would be of utmost clinical and scientific interest. (2) Moreover, studies on the potential effects of binaural beats on the working memory or other cognitive-behavioral functions are quite scarce and highly controversial, not to mention that most of them had assessed the effects of binaural beats *after* the exposure and not during it. (3) There is no study assessing the effects of binaural beats on cognitive-behavioral features simultaneously in both the visuospatial and auditory-verbal modalities; this could allow comparisons of both modalities with each other and develop more comprehensive conclusions or deductions. (4) There is merely one study on the response times; there is no study on the signal detection measures (signal sensitivity and response bias), intrasubject variability of response times, or the BB sound volume effects. And (5) there is no within-subject design with correct, repeated-measures analyses.

The main null hypotheses were the lack of any significant effects of any of the sound interventions as well as short-term training on the hit rate, false alarm rate, working memory, signal detection measures, response times, and intrasubject response time variability in either of the visuospatial or auditory-verbal modalities, in both of them together, and also while assessing the intermodality discrepancies. Additionally, the effects of sex, age, and sound volumes on the cognitive-behavioral parameters of working memory and attention were assessed. There will be qEEG assessments and analyses as well to be reported later.

## 2. Subjects and Methods

### 2.1. Trial Design

This repeated-measures (within-subject) five-arm randomized placebo-controlled clinical trial was performed on 155 experiments in 31 subjects (5 within-subject groups of 31 each). The sample size was determined as 31 subjects based on the few previous studies on the effects of BBs on working memory (e.g., 4, 20, 28, 29, and 34 subjects), noting that a minimum of 20 subjects is recommended for EEG studies [32], and also considering the central limit theorem.

The protocol and/or its ethics were assessed by the institutional review boards of two different institutes (Iran University of Medical Sciences and Institute for Cognitive Science Studies, Tehran, Iran) in accordance with the Helsinki declaration (registration number: IR.IUMS.REC.1399.1353). All subjects were briefed in detail about the methods, goals, and limitations of the study. They filled in and signed written consent forms. Participants could leave the study at will. No changes were made to the methods after the trial commencement.

### 2.2. Pilot Study

Five volunteers were tested with the task in order to evaluate and determine the parameters of the *n*-back task. A pilot EEG study was conducted on a subject as well (to be detailed in the next article). The pilot cases were not included in the sample.

### 2.3. Participants, Eligibility Criteria, and Setting

The subjects were enrolled in the study from different sources including a pool of volunteers registered at the National Brain Mapping Lab, members of online forums, and acquaintances of the first author. The method of sampling was sequential: the subjects were evaluated and enrolled until reaching the desired sample size. In the case of any dropouts, new participants would be acquired. All the experiments were performed in 2021 at the National Brain Mapping Laboratory, Tehran, Iran.

The inclusion criteria were being right-handed healthy subjects aged between 18 and 50 years old, with healthy hearing potential (assessed by Barbara Bates' methods) and with healthy or corrected vision. All the subjects were examined by a physician. The exclusion criteria were the presence of any ongoing or previous clinical neurological or psychiatric diseases (and/or visiting specialists or taking any related medication) and the history of severe head trauma. Furthermore, the included subjects had to fluently know the English numbers 0 to 10.

### 2.4. Preintervention Treatment

On the previous day, a movie of the task was sent to the subject along with instructions on how to play the task. The participant was also instructed to have breakfast. On the experiment day, the subject was seated in a relaxed position in front of a flat computer screen placed about 60 cm away from the subject. The participant put the left index finger on the “a” button of the keyboard and the right index finger on the “l” key. The subject played the *n*-back task for a block of 8 minutes, to become familiarized with the task. They were instructed to pay attention to both the visuospatial and audio-verbal stimuli as much as comfortably possible.

### 2.5. Randomization and Blinding

In this repeated-measures within-subject randomized clinical trial, the subjects were not randomized into any groups, but instead, the order of experiments was randomized and all experiments were performed on each subject. An online digital randomizer was used to randomize the order of interventions in each subject. Random orders were concealed within sequentially numbered containers until interventions were assigned. All randomization steps were done by the first author. The researcher was responsible for playing the audio interventions; therefore, he could not be blinded to the sound interventions. Since the subjects heard the interventions, they were not blinded to the interventions either, whereas they did not know the difference between the rather similar sound interventions (except the silence intervention). Still, we did not consider the study as blinded because of these factors.

### 2.6. Summary of the Study Design

One session sufficed for each patient. Each session had 5 blocks of 8 minutes, with 3-minute rests between every two blocks. In each of the 5 blocks, 3 events happened: (1) the subject played a psychometric task (dual 2-back) for 8 minutes; (2) at the same time, a sound (the intervention) was played in the earphone for 8 minutes; and (3), at the same time, a 32-channel trigger-enabled EEG device recorded the subject's brain activity.

### 2.7. Experimental and Control Sound Interventions

There were 5 “sound interventions” in this study: three binaural beats, a positive control (pure tone), and a negative control intervention (silence, placebo). The binaural beats and pure tone were produced using the Gnaural program (open-source software obtainable from sourceforge.net).

The silence intervention was defined as the absence of any binaural beats or pure tones [4, 16] and not as absolute silence. The binaural beats in use were 10 Hz (the alpha band), 16 Hz (the beta band), and 40 Hz (the gamma band). The base tone of all binaural beats was 240 Hz [4, 16], so that, for example, in the case of the 16 Hz binaural beat, one ear would receive the 240 Hz pure tone, and the other ear would hear 256 Hz pure tone for the 16 Hz BB to be generated in the brain. The left/right ear receiving the base frequency was determined randomly for each subject but remained unchanged for all the interventions of that person. The duration of each intervention was selected as 8 minutes, based on pilot studies. Sound interventions were played immediately before beginning the task and starting the EEG recording and were stopped right after finishing the task and ending the EEG recording. There was a 3-minute rest between every two 8-minute experiments. All the randomized 8-minute interventions of each subject would be carried out in a single session of about an hour (5 blocks of 8 minutes each plus 4 rests of 3 minutes each).

The positive control was the stereo pure tone at 240 Hz, in order to rule out and account for the possible effects of the base frequency. The negative control (i.e., silence) was the lack of any sound interventions; during this placebo intervention, the earphones remained in the ears but no sound (except the task sounds) was played. This was done to rule out the potential placebo effects associated with the experiment setup. Also, this was used as the baseline “condition.”

The loudness of the sound intervention was determined for each subject as the maximum loudness that could be comfortably heard and tolerated by the participant. For each subject, this was adjusted in the beginning; thus, the sound volume was the same for all interventions performed on a given subject. The level of sound intensity was recorded for each participant to be later modeled in statistical analyses. It should be noted that the loudness of the task sound (the auditory-verbal modality of the *n*-back task) was constant and standardized for all subjects and would not be reduced or increased.

The laboratory emphasized keeping a minimum environmental sound noise, e.g., the lab and cell phones would be disconnected and silenced. Still, some mild forms of noise would be inevitable. If some loud noise was accidentally heard at the lab, the session would be discarded and repeated. This happened only once.

### 2.8. Outcomes: Working Memory and Attention Measures

A dual *n*-back task [33] written in Matlab programming language (Mathworks, Natick, Massachusetts, USA) was tested and deemed appropriate for the study. Its parameters were set by the pilot study as *n* = 2 for each modality, 3.330 seconds between every two stimuli (i.e., the duration of each trial), 145 stimuli in each block (i.e., 145 trials per block), lure errors set at 0.2, maximum 40 hits per modality, and the numbers 0 to 10 told by a female voice for the verbal modality. New Matlab code was written by VR to enable the software to also record the response time for each of the modalities.

This task has two modalities that run simultaneously: the visuospatial and auditory-verbal modalities. In each modality, there are 145 short trials during an 8-minute block. Each trial in the visuospatial modality begins at the same time as its counterpart in the verbal modality.

*The visuospatial modality*: in each trial, the visuospatial modality shows a blue square placed randomly in one of the 9 positions of a 3 × 3 matrix (against a black background) for 3.330 seconds. After 3.330 seconds, a new trial begins. The order of the blue square positions has been created in a pseudorandom way; in the beginning of the next trial, the blue square “jumps” to a new random position (or sometimes it remains in the same previous position). This procedure repeats 145 times per block, which lasts about 8 minutes. The subject is instructed to press the “a” key with the index finger of the left hand if the position of the blue square is the same as its position in two trials ago.

*The auditory-verbal modality*: exactly at the same time when the visuospatial modality trial begins, the verbal trial begins as well. A female voice utters a number between 0 and 10. This number has been determined in a pseudorandom manner. After 3.330 seconds, a new trial begins and another number (that may or may not be the same as the previous number) is said. This continues for 145 trials. The subject is instructed to press the “l” key with the right index finger if the number heard in any given trial is the same as the number heard two trials ago.

The *n*-back task has mark trials, in which the stimulus is the same as the stimulus seen or heard in 2 trials ago; the correct response would be to press the key in such mark trials. The appearances of mark trials (when the participant should press the key) on the two modalities were independent of each other, i.e., the sequence of the mark trials in the visuospatial modality had nothing to do with the sequence of the mark trials in the verbal modality. Therefore, sometimes, the mark trials of both modalities could fall within the same trial; in such cases, the subject needed to press both the “a” and “l” keys almost simultaneously.

The *n*-back software collected the trials at which there needed to be responses for each modality (i.e., the mark trials), as well as the trials at which the subject did respond within each modality (i.e., the responses). It also recorded the time between the presentation of the stimulus and pressing the key in each modality.

Based on these data, the hit rates (i.e., sensitivity or true positive rate = the number of true positives / the number of all actual positives) and the false alarm rates (i.e., 1–specificity or false positive rate = the number of false positives / the number of actual negatives) were calculated for each modality. These parameters were calculated once for the whole 8-minute block and once again for the first and second 4-minute halves of each 8-minute block. These calculations were done outside the *n*-back software, using Excel programming (Microsoft, Redmond, Washington, USA).

Each response accompanied immediate feedback: two different strings (related to visuospatial and verbal responses) were written in white font on the bottom of the black screen (left and right sides, respectively). If the response was correct, the relevant string would turn green, and if the response was incorrect, the string would turn red. At the end of each block as well, the subject would be presented with a summary of hits, false alarms (FA), *A*′, and lure errors.

Based on the hit rate and false alarm rate of the whole block and each of the half blocks, two different outcomes were calculated: the working memory capacity was calculated for each modality as (hits–false alarms) × 2 [16, 34]. Signal detection measures were calculated for each modality as *A*′ (showing the subject's sensitivity to the stimulus) and *B*^″^ (showing the subject's response bias (liberal, neutral, and conservative)) [35]. The third outcome was the response time for each modality, which was calculated for the whole block as well as for each of the first and second half blocks. The response time was calculated (for each modality) as the average response time for the block and each of the half blocks. Moreover, the standard deviation (SD) of the response time for the 8-minute block and its 4-minute half blocks was computed. The response time SD was calculated as the measure of intrasubject variability of the response time in each 8-minute block and each half block.

As suggested by Beauchene et al. [4], the difference between outcomes in the second half of each block minus the first half of that block was calculated for 5 of the 7 psychometric parameters, as delta values (e.g., delta working memory capacity or delta response time).

Also, as suggested by another article by Beauchene et al. [16], data pertaining to each subject was ranked among different sessions (for example, working memory scores of each subject were converted to the ranks 1 to 5).

Finally, the discrepancies between the visuospatial and verbal modalities were calculated: For this purpose, each visuospatial parameter was subtracted from the same-name verbal parameter (i.e., the discrepancy = verbal parameter minus visuospatial parameter). This way, a positive discrepancy would indicate a larger verbal parameter compared to its visuospatial counterpart, while a negative discrepancy would point to a greater visuospatial parameter compared to the same-name auditory-verbal parameter. No changes were made to trial outcomes after the trial commencement.

### 2.9. Statistical Analysis

The continuous data were considered normally distributed due to the central limit theorem. Descriptive statistics and 95% confidence intervals (CIs) were computed for all the cognitive/behavioral variables. An unpaired *t*-test was used to compare the mean ages of men and women.

*The primary outcome*: the effects of different sound interventions on cognitive and behavioral variables in each modality (visuospatial or auditory-verbal) were assessed using one- and two-way repeated-measures analyses of (co)variance (ANOVA/ANCOVA). The models were optimized manually. The Mauchly and Levene tests were used to assess the assumptions. In the case of the violation of the sphericity assumption, the Greenhouse-Geisser correction was used. Each significant ANOVA or ANCOVA was followed by a Bonferroni *post hoc* test.

To model and assess both the visuospatial and auditory-verbal modalities simultaneously (and to compare both modalities with each other and to assess the interaction of the intervention by modalities), a mixed-model linear regression was used. For *post hoc* pairwise comparisons following significant regression analyses, the Bonferroni test was used.

For comparing the two halves of each of the five sessions, the delta values (calculated as the outcome in the second session minus the outcome in the first session) were compared with the constant value 0, using a one-sample *t*-test.

The ranked data were compared across the 5 interventions using a Friedman test.

The effects of the interventions on discrepancies between the modalities (calculated as verbal minus visuospatial) were assessed using the ANOVAs, ANCOVAs, and Bonferroni *post hoc* tests. The models were optimized manually.

*The secondary outcomes*: the effects of short-term training (time) were assessed, in a similar fashion to the above analyses: the delta values in different time-blocks were compared with zero. The effects of time on cognitive and behavioral parameters were assessed using manually optimized one- and two-way ANOVAs and ANCOVAs as well as mixed-model linear regressions, all followed by the Bonferroni *post hoc* tests. The ranked data were not assessed over time.

A Pearson correlation coefficient was used to assess the correlations between the response times with the hit rates, false alarm rates, *A*′ indices, and working memories. The level of significance was set at 0.05.

## 3. Results

### 3.1. Participant Flow

After sending online invitations on online forums with about 9000 members and screening the subject pool of the National Brain Mapping Lab, 162 healthy individuals were called and invited to participate in the study. Of them, 58 initially agreed to participate, but 27 were excluded: 19 refused to participate later (mostly because of the fear of COVID-19 cross-infection), 4 were excluded due to neurologic and/or psychiatric conditions not reported originally, 3 were left-handed, and 1 was excluded by the physician due to having cold signs and the possibility of COVID-19 infection (Figure 1). Each of the 5 intervention groups included 31 subjects. Of the 31 participants, 14 were males and 17 were females. The mean (SD) age of the participants in each intervention group was 30.84 ± 6.16 years (range: 19-42). The mean ages of males and females were 31.93 ± 7.08 years (range: 21-42) and 29.94 ± 5.36 years (range: 19-38), respectively. Males and females were not significantly different in terms of mean age (*t*-test, *P* = 0.381). There were no losses or dropouts after the randomization. The trial ended when reaching the desired sample size. No subject complained of any discomforts. No harms were identified with this study.

### 3.2. Effects of the Sound Interventions

Descriptive statistics and 95% CIs for the outcomes in different intervention groups are presented in Tables 1 and 2 and Figures 2–6. The results of the one-sample *t*-test comparing each mean delta value with zero are shown in Tables 1 and 2.

#### 3.2.1. Effects of the Interventions in the Visuospatial Modality

1. *Hit Rate*. The hit rate did not change significantly in different experimental groups (*P* = 0.833). The roles of gender, age, and volume were nonsignificant (*P* ≥ 0.181). Similarly, the interactions were nonsignificant (*P* > 0.2).
2. *False Alarm Rate*. The false alarm rate in different experimental groups did not differ significantly (*P* = 0.607). Sex, age, and sound volume were not significant variables (*P* = 0.172). The interactions were nonsignificant as well (*P* > 0.3).
3. *A*′*(Sensitivity in Signal Detection Theory)*. The *A*′ index did not change significantly across different sound conditions (*P* = 0.832). Sex, age, and sound volume were insignificant (*P* ≥ 0.181). Likewise, the interactions were nonsignificant (*P* > 0.3).
4. *B* ^″^ *(Response Bias in Signal Detection Theory)*. The *B*^″^ index was positive in all experimental groups without any differences across the groups (*P* = 0.179). The effects of gender, age, and sound intensity were nonsignificant (*P* > 0.4). Also, the interaction of age and sound intensity with the experiment was insignificant (*P* ≥ 0.334); however, the gender interaction was significant (*P* = 0.020).
5. *Visuospatial Working Memory*. The working memory capacities were not much different among the sound conditions (*P* = 0.745). The role of sex, age, and sound intensity was nonsignificant (*P* ≥ 0.131). Also, the interactions were nonsignificant (*P* ≥ 0.288).
6. *Reaction Time*. The response speed was faster in the 10 Hz BB group and to a lesser extent in the silence group compared with the other sound conditions (i.e., their response times were shorter than that of the other groups) (*P* = 0.026). The role of age was significant, and age had a direct and positive effect on the response time (*P* = 0.007). Also, the interaction of age and intervention was significant (*P* = 0.045). The Bonferroni test showed no significant pairwise comparison (*P* > 0.5).
7. *Standard Deviation of the Reaction Time*. The SD of response time in the 10 Hz BB group was smaller than that in other groups (*P* = 0.033). The effect of gender was insignificant (*P* = 0.241). But both age (*P* = 0.016) and sound volume (*P* = 0.016) played a significant role; age was directly/positively related to the reaction time SD, but sound volume was inversely related to the reaction time SD. The interactions of gender (*P* = 0.806) and volume (*P* = 0.961) were nonsignificant, but the interaction of age by intervention was significant (*P* = 0.001). The Bonferroni test showed no significant pairwise comparison among the interventions (all *P* values = 1.0).
8. *Delta Hit Rate*. The average visuospatial delta hit rate was negative in all groups, indicating that in the second half of each block, the hit rate decreased compared to the first half. The delta hit rate fluctuated slightly among the different experimental groups in a way the 10 Hz and 40 Hz BB groups had the least drop (*P* = 0.006). The effects of sex and sound intensity were nonsignificant (both *P* values = 0.5). But the sound intensity interaction (*P* = 0.009) was significant, and the sex interaction was marginally significant (*P* = 0.071). The Bonferroni test did not show any significant pairwise comparisons (all *P* values ≥ 0.197).
9. *Delta False Alarm Rate*. All deltas of the average false alarm rates were negative (indicating that the false alarm rate in the second half of each block was lower than that in the first half). No significant differences were observed across the sound conditions (*P* = 0.581). The effects of gender, age, and sound loudness were nonsignificant (*P* ≥ 0.244). The interactions were insignificant as well (*P* ≥ 0.220).
10. *DeltaA*′. The mean ∆*A*′ of most groups was negative, except for the 10 Hz BB group whose delta *A*′ was positive; this indicated that unlike in the other intervention groups, the variable *A*′ increased in the second half of the 10 Hz intervention block compared to its first half. The difference across the conditions was significant (*P* = 0.022). Sex and sound intensity were nonsignificant (*P* ≥ 0.235). The sex interaction was nonsignificant (*P* = 0.224), but the sound intensity interaction was significant (*P* = 0.020). The Bonferroni test showed no significant pairwise comparisons (all *P* values ≥ 0.123).
11. *Delta Working Memory*. The average ∆WM of most groups was negative, except for the 10 Hz BB group whose delta WM was positive, indicating that working memory increased in the second half of the 10 Hz block compared to its first half. The ∆WM varied significantly among the 5 groups (*P* = 0.003). The effects of gender and sound intensity were nonsignificant (*P* > 0.5). The gender interaction was nonsignificant (*P* = 0.242), but the interaction of sound intensity was significant (*P* = 0.004). The Bonferroni test showed no significant pairwise comparisons (all *P* values ≥ 0.141).
12. *Delta Reaction Time*. All mean delta response times were negative, indicating that in the second half of each block, compared to its first half, the response time reduced and the response speed increased. The 5 groups were not different in terms of delta reaction times (*P* = 0.519). The role of age (*P* = 0.536) and its interaction were nonsignificant (*P* = 0.593). The impact of sound volume was significant: louder sounds made the delta response time more positive (*P* = 0.033); however, its interaction was nonsignificant (*P* = 0.878). The role of sex (*P* = 0.951) and the sex interaction were not significant (*P* = 0.382).

#### 3.2.2. Effects of the Interventions in the Auditory-Verbal Modality

1. *Hit Rate*. The hit rate in the 10 Hz BB group was smaller than that of the other groups (*P* = 0.041). The impact of age and sound intensity was insignificant (*P* > 0.3). Similarly, the interactions were nonsignificant (*P* ≥ 0.108). The Bonferroni test showed no significant pairwise comparison (*P* > 0.9).
2. *False Alarm Rate*. The false alarm rate was the highest in the positive control (pure tone) group; the overall difference across the 5 groups was significant (*P* = 0.008). The effects of sex and sound volume were not significant (*P* ≥ 0.150). The sex interaction was nonsignificant (*P* = 0.541). However, sound intensity interaction was significant (*P* = 0.006). No significant pairwise comparison was detected (all *P* values = 1.0).
3. *A*′*(Sensitivity in Signal Detection Theory)*. The *A*′ index varied very subtly among the 5 groups; still, this small difference was statistically significant (*P* = 0.042). This variable was about 1% lower in the 10 Hz BB group, compared to the other groups. The role of sex was marginally significant (*P* = 0.087). The sex interaction was nonsignificant (*P* = 0.818). The impact of sound volume was insignificant (*P* = 0.627), but its interaction was significant (*P* = 0.024). There was no significant pairwise comparison (all *P* values = 1.0).
4. *B* ^″^ *(Bias in Signal Detection Theory)*. All *B*^″^ values were negative in all groups. The difference among the groups was marginally significant (*P* = 0.070). The effects of sex, age, and sound volume were nonsignificant (*P* ≥ 0.45), and so were the interactions (*P* ≥ 0.226).
5. *Verbal Working Memory*. The average verbal WM in the 10 Hz BB group was slightly lower than that of the other groups, and this difference across the 5 groups was marginally significant (*P* = 0.068). The role of sex was marginally significant (*P* = 0.072). The sex interaction was nonsignificant (*P* = 0.901). The role of sound intensity was nonsignificant (*P* = 0.488), but its interaction was significant (*P* = 0.039).
6. *Reaction Time*. There was no significant difference in the speed or time of response to auditory-verbal stimuli in different experimental groups (*P* = 0.405). The effects of sex (*P* = 0.486) and age (*P* = 0.331) were nonsignificant, but the role of sound volume was significant: the louder the sound, the shorter the reaction time (or the faster the response) (*P* = 0.011). The interactions were not significant (*P* > 0.40).
7. *Standard Deviation of the Reaction Time*. The response time SD did not differ significantly across the 5 conditions (*P* = 0.474). The role of sex (*P* = 0.969) and age was nonsignificant (*P* = 0.835). But the sound volume played a significant role: the louder the sound, the less scattered the response time (*P* = 0.018). The interactions were nonsignificant (*P* ≥ 0.213).
8. *Delta Hit Rate*. The mean delta hit rates in the 2 control groups were close to zero, but in the 3 BB groups, they were negative (indicating a relative decrease in the percentage of correct responses in the second half of each group). The difference among the groups was insignificant (*P* = 0.822). The effects of sex, age, and sound volume were nonsignificant (*P* > 0.4). Also, the interactions were nonsignificant (*P* ≥ 0.300).
9. *Delta False Alarm Rate*. All delta false alarm rates were positive, indicating an increase in the percentage of incorrect answers in the second half of each block compared to its first half. The difference across the groups was nonsignificant (*P* = 0.145). The roles of sex, age, sound volume (*P* ≥ 0.144), and the interactions were all insignificant (*P* ≥ 0.09 7).
10. *DeltaA*′. All mean delta *A*′ values were negative, indicating that the *A*′ values decreased in the second half of each block compared to its first half. The groups were not significantly different (*P* = 0.863). The effects of sex, age, sound intensity (*P* ≥ 0.019), and the interactions were all nonsignificant (*P* > 0.6).
11. *Delta Working Memory*. All mean ∆WM values were negative, indicating that verbal working memory in the second half of each block had decreased compared to its first half. The 5 groups were not significantly different (*P* = 0.769). Sex, age, sound volume (*P* ≥ 0.171), and the interactions (*P* > 0.5) were nonsignificant.
12. *Delta Reaction Time*. All auditory-verbal mean delta reaction times were negative, indicating that the reaction time in the second half of each block was slightly shorter than that in the first half. Delta reaction times were not different under the 5 conditions (*P* = 0.572). Age, sex, sound loudness (*P* ≥ 0.334), and the interactions (*P* ≥ 0.301) were insignificant.

#### 3.2.3. Effects of the Interventions in Both Modalities

1. *Hit Rate*. There was no significant difference among the hit rates measured in the 10 groups (5 conditions × 2 modalities, *P* = 0.986). There was a significant difference between the modalities (*P* < 0.0005). The roles of gender (*P* = 0.149), age (*P* = 0.443), and sound volume (*P* = 0.159) were nonsignificant. The interaction of modality by the intervention was nonsignificant (*P* = 0.300).
2. *False Alarm Rate*. Differences in the false alarm rates in different groups were not significant (*P* = 0.632). There was a significant difference between the modalities (*P* < 0.0005). The effects of sex (*P* = 0.165), age (*P* = 0.864), and sound volume (*P* = 0.920) were nonsignificant. The interaction of modality by the intervention was nonsignificant (*P* = 0.930).
3. *A*′. The *A*′ index was not significantly different across the 10 groups (*P* = 0.966). There was no significant difference between the modalities (*P* = 0.612). The impacts of sex (*P* = 0.128), age (*P* = 0.729), and sound volume (*P* = 0.558) were nonsignificant. The interaction of modality by experiment was nonsignificant as well (*P* = 0.481).
4. *B* ^″^. The average *B*^″^ indices were not significantly different across the 10 groups (*P* = 0.833). There was a significant difference between the modalities (*P* < 0.0005). The roles of sex (*P* = 0.944), age (*P* = 0.846), and sound volume (*P* = 0.847) were nonsignificant. Besides, the interaction of modality by experiment was insignificant (*P* = 0.205).
5. *Working Memory*. The working memory capacities were not significantly different among the 10 groups (*P* = 0.931). There was no significant difference between the modalities (*P* = 0.893). The effects of gender (*P* = 0.085), age (*P* = 0.562), and sound volume (*P* = 0.347) were nonsignificant. The interaction of modality by experiment was not significant as well (*P* = 0.422).
6. *Reaction Time*. There was no significant difference in response speed or response time among different groups (*P* = 0.880). There was a significant difference between the modalities (*P* < 0.0005). The role of gender (*P* = 0.923) was nonsignificant, but the effects of age (*P* = 0.036, positive and direct relationship between age and reaction time, *t* = 2.2) and sound volume (*P* = 0.023, an inverse relationship between the sound loudness and reaction time, *t* = −2.4) were significant. The interaction of modality by experiment was insignificant (*P* = 0.388).
7. *Standard Deviation of the Reaction Time*. The SD of response time in different groups was not significantly different (*P* = 0.933). The modalities were significantly different (*P* < 0.0005). The role of sex (*P* = 0.479) and age (*P* = 0.118) was insignificant, but the sound volume (*P* = 0.007, inverse association with reaction time SD, *t* = −2.9) had a significant effect. In addition, the interaction of modality by the intervention was not significant (*P* = 0.843).
8. *Delta Hit Rate*. No significant effect was observed.
9. *Delta False Alarm Rate*. The only significant variable observed was the effect of modality (*P* < 0.0005) in a way that all means of visuospatial delta values were negative (i.e., fewer false responses in the second half compared to the first half) while all means of auditory delta values were positive (i.e., an increase in the rate of incorrect answers in the second half).
10. *DeltaA*′. There was no significant variable.
11. *Delta Working Memory*. No significant variables were detected.
12. *Delta Reaction Time*. There were no significant parameters.

#### 3.2.4. Effects of the Interventions on Ranked Data

No statistically significant Friedman *P* value was observed when comparing the five intervention groups, in terms of the variables: ranked hit rates, ranked false alarm rates, ranked *A*′ indices, ranked working memory capacities, and ranked response times either in the visuospatial modality or in the verbal modality (all *P* values > 0.1).

#### 3.2.5. Effects of the Interventions on the Discrepancies between the Two Modalities

1. *Hit Rate*. The discrepancy between the hit rates in the modalities was almost zero in the 10 Hz group, while in the other groups, the discrepancies were all positive; they were the largest in the silence and 40 Hz groups. The overall difference among the 5 groups was significant (*P* = 0.019). The interaction of intervention by sound was significant (*P* = 0.025), but its interaction by sex was not (*P* = 0.513). The effects of sound volume and sex were insignificant (*P* ≥ 0.471). No significant pairwise comparison was detected by the Bonferroni test (*P* > 0.1).
2. *False Alarm Rate*. The discrepancies between the 2 modalities were all positive; they were almost similar in most groups except in the silence and 40 Hz groups, which showed a higher discrepancy (especially in the 40 Hz group). The overall difference among the groups was significant (*P* = 0.003). The interaction with the sound loudness was significant (*P* = 0.004), but the interaction with sex was not (*P* = 0.560). The effects of sound volume and sex were insignificant (*P* > 0.3). No significant pairwise comparisons were detected (*P* > 0.9).
3. *A*′. In the 10 Hz group, the visuospatial modality had a greater *A*′ index than the verbal modality. In the 16 Hz group, the *A*′ indices were similar in both modalities. In the rest, the verbal *A*′ was greater than its visuospatial counterpart. The overall difference was significant (*P* = 0.014). The interaction with sound volume was significant (*P* = 0.013), but the interaction with sex was not (*P* = 0.684). The effect of sex was marginally significant (*P* = 0.076). The effect of sound volume was insignificant (*P* = 0.411). No significant pairwise comparison was observed (*P* > 0.3).
4. *Working Memory*. The discrepancy was negative in the 10 Hz group, was almost zero in the positive control and the 16 Hz groups, and was positive in the silence and 40 Hz groups (*P* = 0.013). The interaction of sound volume was significant (*P* = 0.012), but the interaction of sex was not (*P* = 0.642). The effects of sound volume and sex were insignificant (*P* > 0.3). No significant pairwise comparison was seen (*P* > 0.3).
5. *Reaction Time*. All discrepancies were positive (verbal response times being longer than the visuospatial response times). The maximum discrepancy was observed in the 10 Hz group, while the least discrepancy was observed in the 16 Hz and 40 Hz BB groups, with a significant overall difference (*P* = 0.019). The interactions with age (*P* = 0.058) and sex (*P* = 0.083) were marginally significant. The effect of age was marginally significant (*P* = 0.065). The effect of sex was insignificant (*P* = 0.258). The only significant pairwise comparison was observed between the 10 Hz group and the 40 Hz group (*P* = 0.048).

### 3.3. Effects of Short-Term Training

Descriptive statistics and 95% CIs for cognitive-behavioral outcomes in different time-blocks are presented in Tables 3 and 4. and Figures 7–11. The results of the one-sample *t*-test comparing each mean delta value with zero are also shown in Tables 3 and 4.

#### 3.3.1. Effects of Training/Time in the Visuospatial Modality

1. *Hit Rate*. The mean hit rate gradually increased over time until it decreased slightly in the last block; this trend was significant (*P* = 0.012). The role of sex was nonsignificant (*P* = 0.243). Furthermore, the interaction of sex by the time variable was nonsignificant (*P* = 0.876). The Bonferroni test showed only a significant pairwise comparison between the first and fourth time-blocks (*P* = 0.037).
2. *False Alarm Rate*. The average false alarm rate gradually decreased until it was almost fixed in the last block, and this trend was significant (*P* = 0.042). The role of sex was nonsignificant (*P* = 0.170). Additionally, the interaction of sex by time was nonsignificant (*P* = 0.480). The Bonferroni test showed no significant pairwise comparison.
3. *A*′*(Sensitivity in Signal Detection Theory)*. The average *A*′ index gradually increased over time until it almost decreased in the last block (*P* < 0.0005). Sex was not significant (*P* = 0.184). The interaction of sex by time was nonsignificant as well (*P* = 0.849). The Bonferroni test showed 3 significant pairwise comparisons between the first and fourth blocks (*P* = 0.001), between the first and fifth blocks (*P* = 0.035), and between the second and fourth blocks (*P* = 0.025).
4. *B* ^″^ *(Bias in Signal Detection Theory)*. The average *B*^″^ index first increased over time and then decreased in the last three blocks (*P* = 0.433). The effects of sex, age, and sound volume were nonsignificant (*P* > 0.4). The interactions were not significant as well (*P* > 0.5).
5. *Visuospatial Working Memory*. The average working memory gradually increased until in the last block, it almost decreased; this trend was significant (*P* < 0.0005). The role of sex (*P* = 0.149) and the interaction of sex by time (*P* = 0.867) were nonsignificant. The Bonferroni test showed 3 significant pairwise comparisons, between the first and fourth time-blocks (*P* = 0.001), between the first and fifth blocks (*P* = 0.023), and between the second and fourth blocks (*P* = 0.011).
6. *Reaction Time*. The speed of response gradually increased (or the reaction time decreased over time); this trend was significant (*P* < 0.0005). The role of sex was insignificant (*P* = 0.914). Also, the interaction of sex and time was insignificant (*P* = 0.817). The Bonferroni test showed 4 significant pairwise comparisons: between the first and fourth time-blocks (*P* = 0.003), between the first and fifth blocks (*P* < 0.0005), between the second and fourth blocks (*P* = 0.010), and between the second and fifth blocks (*P* < 0.0005).
7. *Standard Deviation of the Reaction Time*. The SD of response time in the first two blocks was almost constant and then gradually decreased until in the last block, it increased; this trend was significant (*P* = 0.045). The effect of sex was insignificant (*P* = 0.241). But both the variables age (*P* = 0.016) and sound volume (*P* = 0.016) played a significant role. In addition, the interactions were nonsignificant (*P* > 0.2). The Bonferroni test showed no significant pairwise comparison (all *P* values > 0.6).
8. *Delta Hit Rate*. The delta hit rate fluctuated slightly and only marginally significantly (*P* = 0.084). The role of sex (*P* = 0.474) and the sex-by-time interaction were not significant (*P* = 0.839).
9. *Delta False Alarm Rate*. It fluctuated significantly over time (*P* = 0.015). The role of sex was nonsignificant (*P* = 0.603). The interaction of sex by time was nonsignificant as well (*P* = 0.739). The Bonferroni test showed a significant pairwise comparison between the second and fourth blocks (*P* = 0.011).
10. *DeltaA*′. ∆*A*′ did not fluctuate significantly over time (*P* = 0.108). The role of sex was nonsignificant (*P* = 0.222). Similarly, the interaction of sex and time was insignificant (*P* = 0.730).
11. *Delta Working Memory*. Most of the mean ∆WM values were negative, indicating that the working memory capacity in the second half of each block was slightly smaller than that in the first half. ∆WM fluctuated significantly over time (*P* = 0.025). The role of sex was nonsignificant (*P* = 0.568). Likewise, the interaction of sex and time was nonsignificant (*P* = 0.692). The Bonferroni test showed no significant pairwise comparisons (*P* values ≥ 0.059).
12. *Delta Reaction Time*. Most of the mean delta response time values were negative, indicating that the reaction time in the second half of each block was slightly shorter than the reaction time in the first half (i.e., the reaction speed increased slightly in the second half). The delta response time did not change significantly over time (*P* = 0.090). The role of age (*P* = 0.343) and its interaction with time (*P* = 0.368) were not significant. The role of sound volume was significant (*P* = 0.030). But its interaction was nonsignificant (*P* = 0.161).

#### 3.3.2. Effects of Training in the Auditory-Verbal Modality

1. *Hit Rate*. The average hit rate gradually increased until it almost became constant in the third and fourth blocks and then decreased slightly in the last block; this trend was significant (*P* = 0.006). The role of sex was insignificant (*P* = 0.241). Also, the interaction of sex and time was insignificant (*P* = 0.791). The Bonferroni test showed only a significant pairwise comparison between the first and fourth blocks (*P* = 0.003).
2. *False Alarm Rate*. The average false alarm rate decreased gradually over time, but this trend was not significant (*P* = 0.412). The roles of sex (*P* = 0.167), age (*P* = 0.953), and sound volume (*P* = 0.983) as well as the interactions of time by sex (*P* = 0.116), age (*P* = 0.330), and sound volume (*P* = 0.656) were insignificant.
3. *A*′*(Sensitivity in Signal Detection Theory)*. The average *A*′ index gradually increased until in the last block, it decreased slightly (*P* = 0.003). The role of sex was marginally significant (*P* = 0.077). The interaction of sex and time was not significant (*P* = 0.866). The Bonferroni test showed a significant pairwise comparison between the first and fourth blocks (*P* = 0.002).
4. *B* ^″^ *(Bias in Signal Detection Theory)*. The average *B*^″^ did not change significantly over time (*P* = 0.223). The roles of sex (*P* = 0.471), age (*P* = 0.983), and sound volume (*P* = 0.594) and the interactions were nonsignificant (*P* > 0.26).
5. *Verbal Working Memory*. The average auditory-verbal WM gradually increased until it reached a plateau in the last block (*P* = 0.001). The role of sex was marginally significant (*P* = 0.063). The interaction of sex and time was insignificant (*P* = 0.822). The Bonferroni test showed 2 significant pairwise comparisons between the first and third blocks (*P* = 0.033) and between the first and fourth blocks (*P* = 0.002); the comparison between the first and fifth blocks was marginally significant (*P* = 0.062).
6. *Reaction Time*. The speed of response increased significantly over time, i.e., the average response time decreased by training (*P* = 0.003). The roles of sex (*P* = 0.486) and age (*P* = 0.331) were nonsignificant, but the role of sound volume was significant (*P* = 0.011). The interactions of time by sex (*P* = 0.110) and sound volume (*P* = 0.404) were insignificant, although the interaction of age by time was significant (*P* = 0.048). The Bonferroni test showed 5 significant pairwise comparisons between the first and third blocks (*P* = 0.005), the first and fourth (*P* < 0.0005), the first and fifth (*P* < 0.0005), the second and fourth (*P* = 0.013), and the second and fifth blocks (*P* = 0.010).
7. *Standard Deviation of the Reaction Time*. The SD of auditory-verbal response time was at first almost constant and even slightly increasing, but then, it decreased from the third block onwards (*P* = 0.031). The roles of sex (*P* = 0.969) and age (*P* = 0.835) were insignificant. But the sound volume played a significant role (*P* = 0.018). The interactions were nonsignificant: age (*P* = 0.091), volume (*P* = 0.151), and sex (*P* = 0.165). No significant pairwise comparison was detected (*P* values > 0.2).
8. *Delta Hit Rate*. The mean delta hit rate did not change significantly over time (*P* = 0.643). Sex, age, sound intensity (*P* ≥ 0.441), and the interactions were nonsignificant (*P* ≥ 0.162).
9. *Delta False Alarm Rate*. No significant changes were observed (*P* = 0.083). The effects of sex, age, and sound loudness were nonsignificant (*P* ≥ 0.144). Also, the interactions were nonsignificant (*P* = 0.253).
10. *DeltaA*′. The mean ∆*A*′ did not change significantly over time (*P* = 0.306). Sex, age, sound intensity (*P* ≥ 0.019), and the interactions were insignificant (*P* ≥ 0.146).
11. *Delta Working Memory*. The mean ∆WM did not change significantly (*P* = 0.280). The role of sex, age, and sound volume was nonsignificant (*P* ≥ 0.171). Also, the interactions were nonsignificant (*P* ≥ 0.177).
12. *Delta Reaction Time*. The mean delta of auditory-verbal response time did not change significantly over time (*P* = 0.452). The role of age, sex, and sound loudness (*P* ≥ 0.334), and also, their interactions by the time variable were nonsignificant (*P* ≥ 0.170).

#### 3.3.3. Effects of Training in Both Modalities

1. *Hit Rate*. The mean hit rate gradually increased until it began to decrease slightly in the last block (*P* < 0.0005). There was a significant difference between the 2 modalities (*P* < 0.0005). The effects of sex (*P* = 0.149), age (*P* = 0.443), and sound volume (*P* = 0.159) were nonsignificant. Also, the interaction of modality and time was nonsignificant (*P* = 0.645). The Bonferroni test showed 2 significant pairwise comparisons, between the first and fourth time-blocks (*P* = 0.001) and between the first and fifth time-blocks (*P* = 0.008).
2. *False Alarm Rate*. The average false alarm rate gradually decreased until it became rather fixed in the last block (*P* = 0.013). There was a significant difference between the 2 modalities (*P* < 0.0005). The roles of sex (*P* = 0.165), age (*P* = 0.864), and sound volume (*P* = 0.920) were nonsignificant. Additionally, the interaction of modality and time was nonsignificant (*P* = 0.654). The Bonferroni test showed two significant pairwise comparisons, between the first and fourth time-blocks (*P* = 0.054) and between the first and fifth blocks (*P* = 0.012).
3. *A*′*(Sensitivity in Signal Detection Theory)*. The average *A*′ gradually increases over time until it almost decreases in the last block (*P* < 0.0005). There was no significant difference between the modalities (*P* = 0.594). The effects of sex (*P* = 0.128), sound volume (*P* = 0.558), and age (*P* = 0.729) were nonsignificant. Also, the interaction of modality and time was nonsignificant (*P* = 0.579). The Bonferroni test showed 4 significant pairwise comparisons, between the first and third time-blocks (*P* = 0.040), between the first and fourth time-blocks (*P* < 0.0005), between the first and fifth blocks (value *P* < 0.0005), and between the second and fourth blocks (*P* = 0.033).
4. *B* ^″^ *(Bias in Signal Detection Theory)*. The average *B*^″^ value did not change significantly over time (*P* = 0.378). There was a significant difference between the modalities (*P* < 0.0005). The roles of sex (*P* = 0.946), age (*P* = 0.847), and sound volume (*P* = 0.848) were nonsignificant. Also, the interaction of modality and time was insignificant (*P* = 0.430).
5. *Working Memory*. The average working memory gradually increased until it almost decreased in the last session (*P* < 0.0005). There was no significant difference between the modalities (*P* = 0.887). The role of sex (*P* = 0.085), age (*P* = 0.562), and sound volume (*P* = 0.347) was not significant. Similarly, the interaction of modality and time was nonsignificant (*P* = 0.455). The Bonferroni test showed 4 significant pairwise comparisons, between the first and third time-blocks (*P* = 0.009), between the first and fourth time-blocks (*P* < 0.0005), between the first and fifth blocks (value *P* < 0.0005), and between the second and fourth blocks (*P* = 0.018).
6. *Reaction Time*. The speed of response constantly increased over time, i.e., the average reaction time decreased (*P* < 0.0005). There was a significant difference between the modalities (*P* < 0.0005). Sex (*P* = 0.923) was nonsignificant, but age (*P* = 0.036, a positive relationship with reaction time, *t* = 2.2) and sound volume (*P* = 0.023, an inverse association with reaction time, *t* = −2.4) were significant predictors. The interaction of modality and time was not significant (*P* = 0.964). The Bonferroni test showed 5 significant pairwise comparisons, between the first and third sessions (*P* = 0.010), between the first and fourth sessions (*P* < 0.0005), between the first and fifth sessions (*P* < 0.0005), between the second and fourth sessions (*P* = 0.002), and between the second and fifth sessions (*P* < 0.0005).
7. *Standard Deviation of the Reaction Time*. The average SD of response time in the first two blocks was almost constant, and then, it gradually decreased until it increased in the last block; this trend was significant (*P* = 0.017). There was a significant difference between the 2 modalities (*P* < 0.0005). The effects of sex (*P* = 0.479) and age (*P* = 0.118) were nonsignificant, but the sound loudness (*P* = 0.007, an inverse relationship, *t* = −2.9) was significant. The interaction of modality and time was nonsignificant (*P* = 0.964). The Bonferroni test showed no significant pairwise comparison (*P* > 0.18).
8. *Delta Hit Rate*. No significant variables were observed.
9. *Delta False Alarm Rate*. All variables were nonsignificant except for the role of modality (*P* < 0.0005) and the interaction of modality by time (*P* = 0.006).
10. *DeltaA*′. No variables had a significant role.
11. *Delta Working Memory*. No significant variables were detected.
12. *Delta Reaction Time*. There was no significant variable.

#### 3.3.4. Effects of Training on the Discrepancies between the Two Modalities

1. *Hit Rate*. All discrepancies were positive. No significant variable was observed in the 3-way repeated-measures ANCOVA.
2. *False Alarm Rate*. All FA discrepancy means were positive. There was no significant variable.
3. *A*′. The *A*′ discrepancy means revolved around zero, without any significant variable.
4. *Working Memory*. The WM discrepancy averages were close to zero, without any significant variable.
5. *Reaction Time*. All discrepancies were positive, without any significant difference.

### 3.4. Correlations between Response Times with Cognitive Functions

The Pearson correlation coefficient showed significant negative correlations between response times and the variables hit rate, *A*′, and working memory in many sessions; it also found significant positive correlations between response times and false alarm rates in some sessions (Tables 5 and 6).

## 4. Discussion

Since many of the variables studied by us were not available in the literature on binaural beat stimulation effects, we were limited to comparing and discussing those aspects with studies from other fields that had similar concerns. The assessment of visuospatial deltas in the present study showed that the mean delta of visuospatial hit rate in all groups was negative indicating that in the second half of each session, the hit rate decreased compared to the first half. This negativity might be due to fatigue or boredom. The extent of this decrease in the 10 Hz group was significantly less than that in the other groups. This means that the alpha band might counterbalance mechanisms underlying fatigue in the second half through a possible range of hypothetical mechanisms such as increasing the concentration or reducing fatigue. Also, the mean deltas of visuospatial *A*′ as well as visuospatial spatial working memory were negative in most groups, except for the 10 Hz BB group whose delta values were positive, indicating that the variables visuospatial *A*′ and working memory increased in the second half of the 10 Hz block relative to its first half—and these differences among the groups were significant. Our findings in terms of suitability of alpha-band binaural beats (in the visuospatial modality) were in line with another study comparing 9.55 Hz binaural beats versus control [30]. On other cognitive domains, some studies have also shown favorable results concerning alpha binaural beats: a study showed improvements in Stroop test performance as a result of 10.2 Hz binaural beat stimulation [36]. Another research showed that 8 weeks of entraining the brain using a rhythmic audiovisual stimulator at 10 and 18 Hz would improve the IQ and memory of children with disabilities [37]. McMurray [38] showed that brain stimulation with alpha binaural beats may improve both attention and working memory in healthy elderly who may naturally experience decreased alpha activity. Higher amplitudes of alpha brain waves might be associated with improved working memory, attention, vigilance, information processing speed, perceptual abilities, and inhibitory processes [23, 30, 39–44]. Improved visual working memory has been linked to increased alpha rhythms [44]. Perhaps, alpha oscillations may indirectly improve working memory by filtering out irrelevant information and averting disturbances caused by conflicting stimuli [45–47]. Nevertheless, not all results are in favor of the alpha stimulation: Beauchene et al. [4, 16] failed to find any effects of 5 minutes of alpha BB stimulation on visuospatial or verbal working memories. More interestingly, Wahbeh et al. [23] asserted that 30 minutes of alpha binaural beat stimulation might deteriorate auditory-verbal learning. Their results were in line with another finding of the present study: in the auditory-verbal modality, we observed that the hit rate and the auditory *A*′ were slightly but statistically significantly lower in the 10 Hz BB group than the other groups (especially compared to the silence and 40 Hz groups). This pattern was also seen in verbal working memory, even though in only a marginally significant way. Although more research is needed for confident interpretation of our findings, it seems that perhaps the alpha binaural beat stimulation can improve visuospatial working memory at the expense of deteriorating verbal working memory, possibly by shifting the attention and/or allocating cognitive resources to the visuospatial modality. Future research simultaneously performed on both the visuospatial and verbal modalities is needed to verify our results. Our finding in terms of delta values in the visuospatial modality contrasted with the only other study that had used the delta method: Beauchene et al. [4] compared delta visuospatial accuracies among control interventions as well as 5 Hz, 10 Hz, and 15 Hz binaural beats. They found that delta accuracy values were negative in all groups, except in their 15 Hz group, which had a positive delta accuracy [4]. Unlike the present study, in their study, the 10 Hz intervention caused one of the largest negative visuospatial delta accuracies [4]. The difference observed between the results of the two studies needs more research for possible explanations. It might be speculated that the lack of any rest between sessions as well as shorter durations of sessions in their study [4] might change the fatigue states of subjects, compared to our research. Moreover, for calculating delta values, they omitted 2 middle minutes of each session and subtracted the last 1.5 minutes from the first 1.5 minutes (while we subtracted the second half from the first half in order to avoid data loss). In the verbal modality of the present study, the false alarm rate was slightly but statistically significantly higher in the pure tone and 40 Hz groups, while it was the minimum in the silence and 10 Hz groups. Without any similar articles, we cannot compare and discuss this more. It is suggested that some binaural beats can entrain brain waves [20–22, 24] and alter the functioning of the reticular formation (responsible for the regulation of arousal, attention, concentration, and vigilance) [23]. Although our study focused on working memory, the *A*′ and *B*^″^ indices were a part of the signal detection theory, which has been associated with attention as well [48, 49]. Attention acts like a filter that oversees information and picks a limited amount of it to allow locking on goal-related stimuli and discarding undesired ones [50]. Enhancing this important gateway to information can improve many other cognitive processes as well [51–53]. Working memory is heavily interlaced with attention [53, 54], and binaural beats might improve attention (although studies are controversial and a few): Colzato et al. [55] assessed the effects of 40 Hz binaural beats versus a constant tone (as control) on attention measured by a global-local task. They concluded that binaural beats might not induce suppression of task-irrelevant information but can condense the spotlight of attention [55]. Crespo et al. [56] assessed the effects of listening to 20 minutes of theta and beta binaural beats on attention; they did not observe any changes in the attention or the EEG activity of participants [56]. Kennel et al. [57] investigated whether listening to 9 sessions of 20-minute beta binaural beats during 3 weeks could reduce inattention in children with attention-deficit/hyperactivity disorder. They did not find any significant result [57]. On the other hand, another study found some positive effects of beta binaural beats on attention [20].

Unlike Beauchene et al. [16] who asserted that there was a significant increase in *ranked* working memory in their 15 Hz group, we could not find any effect of binaural beats on any ranked working memory or response time measures in either modality. The reason for the dispute can be in methodological differences such as durations of stimulations, frequencies used (5, 10, and 15 in their study versus 10, 16, and 40 in ours), and statistical analyses. Beauchene et al. [16] used a between-subject analysis that is always used for the comparison of 2 groups (a Mann–Whitney *U* test) for comparing 6 within-subject (repeated-measures) groups. No other studies had ranked their findings so that we can compare our results with them.

In this study, response times were negatively correlated with the hit rates, *A*′ indices, and working memories, while they were positively correlated with false alarm rates. This is in line with previous findings [58]. In our study, response times were shorter in the visuospatial modality compared to the auditory-verbal modality even though the verbal modality responses had been done with the dominant hand. This contrasted with the literature which indicated that auditory-verbal responses may be faster than visuospatial responses; it also was contrary to the literature indicating that those responses entered with the dominant hand may be faster [59–61]. Possible reasons for our findings might be the much longer duration of the visual stimulus compared to the verbal one, as well as a probable preference of the individuals to pay more attention to the visuospatial modality; also perhaps, the subjects considered the visuospatial modality as the dominant modality (as also indicated by their *B*^″^ indices). Also, other methodological specifications such as the setup of the current study and the simultaneous exposure of the subjects to both the visuospatial and auditory-verbal stimuli in this study might play a role. Response times are a function of factors such as sex, although this is controversial with many studies not finding a difference and one finding a difference merely in right-handed individuals [59, 60, 62–64]; also, age [60, 62, 63], limb dominance [59, 60], practice [65–67], and properties of stimulus such as duration or intensity [61] might predict the response time. Attention as well might affect the speed of responses, especially the complicated ones [61, 68, 69]. Standard deviations of reaction times can be associated with intelligence [69]. We did not observe a link between the reaction time and sex but found aging to have a significant role. Interestingly, despite the lack of improvement in cognitive indices in this study (such as attention indicated by the *A*′ index and working memory) after the third or four sessions, response times continued to become shorter and shorter by training until the last session, which can imply the effect of practicing on reaction time [67].

In the visuospatial modality, the response time to the visual stimulus showed a significant decrease in the 10 Hz group compared to the other groups (especially compared to the 16 Hz and pure tone groups). There was only one study regarding the effects of binaural beats on response times: Beauchene et al. [16] observed no significant difference between response times measured under 5 Hz, 10 Hz, and 15 Hz binaural beats compared to controls. The difference between their and our findings might stem from different methodologies such as dissimilar durations of sessions, different modalities in question (visuospatial in this study versus verbal in theirs), and statistical analyses; for instance, they used the between-subject 2-group Mann–Whitney *U* test for comparing 6 repeated-measures (within-subject) groups, which was not correct. Furthermore, it should be noted that like in their study (which used the verbal modality), we as well did not observe any significant effect of binaural beats on the response time in the verbal modality. It was observed in the current study that a person's age had a significant effect on response times (i.e., with increasing age, the speed of reaction decreased). It was also observed that the intrasubject variability of the visuospatial reaction time was slightly smaller in the 10 Hz group than in the other groups. This variability of reaction time increased in older people and also increased with decreasing the sound intervention volume. The effects of age on response times have been documented earlier [60, 62, 63]. The effect of the intervention volume on reaction time variability might imply that these interventions could have played a positive role in decreasing the intrasubject variability, perhaps through masking and reducing potential auditory distractions existing in the lab environment. No other study has assessed this item. Louder sounds also made the visuospatial delta response times more positive, meaning that by hearing louder sounds, the reactions became slower (longer response times) in the second half of each 8-minute session compared to its first half. Perhaps, louder sounds might have some exhausting effects, but no studies have ever assessed this factor, and without further evidence, we cannot confidently interpret the results. In the auditory-verbal modality, increasing the volume of the audio intervention could accelerate the response and reduce the reaction time as well as the intrasubject variability of reaction times. This again might be a result of the intervention sounds masking potential auditory distractors; nevertheless, this is not the only possible hypothetical explanation. For instance, it is shown that increasing the volume of background noise can intensify alpha brainwaves and reduce the power of beta rhythms [70]. Moreover, there might be some generic effect to all the tested interventions (including pure tone); for example, white noise might improve learning [71].

The comparison of modalities with each other showed that both the hit and false alarm rates in the auditory-verbal modality were greater than those in the visuospatial modality. This indicated the tendency of participants to respond to auditory-verbal stimuli more freely and more frequently. Still, the working memory capacities and *A*′ indices remained similar in both modalities. The mean values of the *B*^″^ index in the visuospatial modality were positive, whereas in the auditory-verbal modality, these values were negative. This suggests that the individuals' biases in the auditory-verbal modality were *liberal* and to some extent neutral in some groups, implying a degree of tendency to respond to auditory stimuli with the least skepticism and when feeling the slightest sense of familiarity. On the other hand, in the visuospatial modality, the subjects' biases were *conservative*, meaning that they did not respond to the visuospatial stimuli unless being rather confident. These biases were not affected by the 5 sound interventions. It was also found that the reaction time in the visuospatial modality was shorter than the reaction time in the auditory-verbal modality. Instead, the intrasubject variability of reaction time was greater in the visuospatial modality than that in the auditory-verbal modality. Aging and decreasing the sound volume could slow down the response, while decreasing the loudness of the sound could increase the variability of the reaction time.

Another interesting point found in the comparison of the modalities was that all the average visuospatial delta FA rates were negative (i.e., there were fewer incorrect answers in the second half compared to the first half), whereas all the mean verbal delta FA rates were positive (more incorrect responses in the second half). This indicated that during an 8-minute session, the efficacy reduces in the auditory-verbal modality while it improves in the visual modality. Such a simultaneous change in both modalities might be interpreted as shifting one's attention (or other cognitive resources such as error detection) from the auditory-verbal modality to the visuospatial one. The 5 audio interventions did not play a role in these patterns. However, when we calculated the differences between both modalities in terms of cognitive-behavioral parameters, the audio interventions seemed to play a significant role in many intermodality discrepancies: In the case of hit rate, interestingly, two inverse patterns were observed in both modalities, resulting in the maximum intermodality discrepancies in the silence or 40 Hz groups, and the minimum discrepancy in the 10 Hz group (which showed the highest visuospatial hit rate and the lowest verbal hit rate). An almost similar pattern was observed in the false alarm rates, causing the greatest and smallest discrepancies in the 40 Hz and 10 Hz groups, respectively. Working memory and the *A*′ index almost followed a similar pattern to the hit rate, with the silence and 40 Hz groups having the highest positive discrepancies and the 10 Hz group having a negative discrepancy—indicating a greater visuospatial *A*′ compared to the verbal *A*′, in the 10 Hz group. The average response time was always longer in the verbal modality compared to the visuospatial one. In the verbal modality, it was the slowest (longest) in the 10 Hz group and the fastest (shortest) in the 40 Hz group; this was inverse in the visuospatial modality, being the fastest in the 10 Hz group. As a result, the discrepancy was the maximum in the 10 Hz group, which was significantly greater than that seen in the 40 Hz group. It seems that the assessed audio interventions can have different (and perhaps inverse) effects on the two modalities. The closest study to our design may be that of Hommel et al. [72] who assessed the impact of 40 Hz binaural beats on the cross-talk of two tasks. Originally, lower frequencies of binaural beats used to be associated with mental relaxation while higher frequencies were thought to induce attentional concentration and alertness [73, 74]. Accordingly, high-frequency beats were expected to bias the cognitive control toward focus and persistence, i.e., more attentional resources to be assigned to the task at hand [72]. However, some recent findings contradicted this anticipation: Reedijk et al. [75] compared the effects of the alpha and gamma binaural beat stimulations on subjects' performance in an attentional blink [76] task, which presents subjects with two visual targets in a stream of stimuli. If the second target is presented briefly after the first, participants usually miss the second one. This has been linked to overcontrol, which is an excessively strong focus on the first target, leaving too few resources for the second one [77]. Reedijk et al. [75] observed that the alpha stimulation did not affect attentional blink, whereas the gamma entrainment decreased the attentional blink, suggesting that, unlike the original expectation, gamma stimulations might broaden the distribution of available focus (instead of inducing a stronger focus). Another study of Reedijk et al. [78] might suggest the same: they reported that the gamma stimulation might improve performance in a divergent (but not in a convergent) thinking task, perhaps because divergent thinking may benefit more from broadly distributed resources compared to convergent thinking [72]. The dual *n*-back task used in our study needs divided attention, and therefore, it might also benefit from a broader distribution of attentional and cognitive resources. Thus, perhaps the discrepancy observed between the response times in the two modalities can be considered a marker of the distribution of cognitive resources, i.e., flexibility. From the *B*^″^ indices and response times, it can be speculated that the dominant modality (the one taking more attentional resources) may have been the visuospatial one. From the combination of significant intermodality discrepancies, it might be suggested that the 40 Hz intervention, silence, and to a lesser extent the 16 Hz and pure tone interventions could shift more resources to the verbal modality, increasing cognitive flexibility as seen by the increased hit rates, FA rates, *A*′ indices, working memories, and faster responses in the verbal modality (and the reverse outcomes in the visuospatial modality). On the other hand, the 10 Hz intervention might shift the attentional resources to the visuospatial modality, increasing cognitive persistence—indicated by the faster responses and increased hit rates, *A*′ indices, and working memories in the visuospatial modality. Although our findings were in line with the three studies on cognitive flexibility [72, 75, 78], future studies are warranted to assess our speculation.

The findings of this study showed that short-term training could affect a person's cognitive function, such that some cognitive parameters improved over the 40-minute time of this study (e.g., reaction time); some others usually improved until the third or fourth sessions and then either reached a plateau or slightly decreased (e.g., working memory). There is a capacity limit on the number of chunks concurrently retained in working memory (somewhere between one and four) [3–8]. Naturally, working memory has been thought of as a permanent feature correlated with fluid/general intelligence [79–81] that seems to be highly heritable [82] and resistant to extraneous experiences [83]. Nevertheless, recent evidence suggests otherwise, that working memory can be enhanced by medication or practice [3, 84, 85], although not all recent studies agree with the malleability of working memory [86]. A study using a dual *n*-back task showed that training can improve test results as well as general fluid intelligence [87]. Dual-task performance may be improved with dual-task training and repetition plus tasks like dual *n*-back that may activate the right dorsolateral prefrontal cortex [88, 89]. Our findings showed that short-term training can be useful to some extent, but after some sessions, the tendency to improve reduces; this is perhaps a result of fatigue [90] or simply because some limits might have been reached. Notably, practicing a working memory task might not be necessarily transferable to other tasks [91]. Interestingly, training did not affect discrepancies between the modalities. No studies were available to compare our results with.

### 4.1. Limitations and Advantages

This study was limited by some factors. Like all previous studies regarding the effects of binaural beats on working memory, no *a priori* power calculations were done to determine the sample size in this study. Still, the current sample size (*n* = 155 trials in 5 groups of 31 each) was comparable to or larger than most of the few articles in this field and also provided adequate powers to calculate numerous significant results. Furthermore, since the *n*-back task seems to require upholding, continuous updating, and processing of information, it has face validity as a working memory task [92]; however, recent evidence casts doubt on its construct validity as a working memory task, as it might measure attention as well, especially in older subjects [92]. Moreover, interpreting *n*-back findings needs utmost care [93]. This is why we explicitly evaluated *n*-back results and also calculated not accuracy and reaction latency, but instead the hit and false alarm rates as well as *A*′ and *B*^″^ indices besides response times and intrasubject response time variabilities, as recommended earlier [93]. An advantage over previous studies is that we assessed both the visuospatial and auditory-verbal modalities simultaneously. This allowed us to observe that the significant improvement detected in visuospatial working memory might actually occur at the cost of a decline in verbal working memory and that the bigger picture might be indicative of some shifts of attention or allocated resources between the modalities. On the other hand, we controlled for numerous confounding variables such as IQ and even genetics by adopting a within-subject design. The generalizability of our findings is limited to right-handed healthy adults and young adults. Still, it benefited from a rather broad age range and various intervention sound volumes.

## 5. Conclusions

Within the limitations of this randomized clinical trial on the alteration of working memory and attention measures under the effect of binaural beats, it could be concluded that

1. in the visuospatial modality, the alpha binaural beat stimulation was able to accelerate reactions and reduce response latencies as well as intrasubject variabilities of reaction times. The 10 Hz BB entrainment could also change the pattern of decline in some visuospatial parameters over time (indicated by delta values): this intervention reduced or stopped the extent of decline over time in terms of visuospatial working memory, *A*′, and hit rate. Aging might slow down responding to the stimulus and increase the intrasubject variability of reaction time. This reaction time variability increased also with decreasing the sound intervention volume. By listening to louder sounds, reactions might become slower after some time (indicated by visuospatial delta response times becoming more positive under louder sounds).
2. In the auditory-verbal modality, the 10 Hz intervention reduced *A*′, hit rate, and false alarm rate (compared to all groups except silence). Working memory was as well reduced by the 10 Hz BB, but only in a marginally significant way. Louder sounds might accelerate responses and reduce intrasubject variabilities of reaction times.
3. The audio interventions could as well affect the discrepancies between the two modalities: the intermodality discrepancies in the hit rates were the lowest in the 10 Hz group and the greatest in the silence and 40 Hz groups. Similarly, the minimum and maximum false alarm rate discrepancies were observed in the 10 Hz and 40 Hz groups, respectively. In the case of working memories and *A*′ indices, the 10 Hz intervention caused a negative discrepancy (indicating a greater working memory and *A*′ in the visuospatial domain than the verbal one) while the other interventions caused positive or almost-zero discrepancies, with the silence and 40 Hz interventions causing the highest positive discrepancies. The 10 Hz entrainment caused the greatest intermodality discrepancy of response time while the 40 Hz stimulation caused the smallest response time discrepancy.
4. Each of the parameters working memory or *A*′ index was rather similar in the visuospatial versus verbal modalities, while both the hit and false alarm rates were greater in the auditory-verbal modality compared to the visuospatial one.
5. Response biases (the *B*^″^ indices of the signal detection theory) indicated that in the auditory-verbal modality, the participants mostly had a liberal bias (implying their tendency to respond to auditory stimuli with minimum hesitation) and in some groups somehow a neutral bias in the auditory-verbal modality. Instead, in the visuospatial modality, the subjects had conservative biases, implying that they would not respond to visuospatial stimuli unless being reasonably certain about it.
6. While in the visuospatial modality, mean delta false alarm rates were negative (indicating fewer errors in the second half of each 8-minute block); they were positive in the auditory-verbal modality (indicating more errors in the second half). This might imply a shift of attention and/or cognitive resources to the visuospatial modality over time.
7. Response times were shorter in the visuospatial modality than in the auditory-verbal one. However, the intrasubject variability of reaction times was smaller in the auditory-verbal modality than in the visuospatial one.
8. Faster reactions may accompany better hit rates, working memories, and *A*′ indices, as well as lower false alarm rates.
9. Regardless of the modality, aging and reduced intervention sound volume may slow down the response (and increase response times). Reduced sound intensities may as well increase the intrasubject variability of response times.
10. Short-term training can improve the hit rate, false alarm rate, working memory, *A*′ index, and response time.

## Figures and Tables

**Figure 1:** The flow diagram of the interventions randomized within 31 participants.

**Figure 2:** Mean and 95% CIs for the hit rates and false alarm rates in each of the 2 modalities, and in the sexes, under the effect of 5 different interventions.

**Figure 3:** Mean and 95% CIs for the parameters *A*′ (sensitivity) and *B*^″^ (response bias) in each of the modalities and in the sexes, in 5 intervention groups.

**Figure 4:** Mean and 95% CIs for the response time and intrasubject response time variability in the modalities and in the sexes, in different intervention groups.

**Figure 5:** Mean and 95% CIs for delta hit rates, delta false alarm rates, and delta *A*′ (sensitivity) in each of the 2 modalities and in the sexes, under various sound conditions.

**Figure 6:** Mean and 95% CIs for delta working memory and delta response time in each of the modalities and in the sexes, in 5 sound groups.

**Figure 7:** Mean and 95% CIs for the hit rates and false alarm rates in each of the 2 modalities and in the sexes, in different time-blocks.

**Figure 8:** Mean and 95% CIs for the parameters *A*′ (sensitivity) and *B*^″^ (response bias) in the modalities, sexes, and time-blocks.

**Figure 9:** Mean and 95% CIs for the response time and intrasubject response time variability in the modalities, sexes, and time-blocks.

**Figure 10:** Mean and 95% CIs for delta hit rates, delta false alarm rates, and delta *A*′ (sensitivity) in each of the modalities, sexes, and different time-blocks.

**Figure 11:** Mean and 95% CIs for delta working memory and delta response time in each of the 2 modalities, in women and men, in different time-blocks.

**Table 1:** Descriptive statistics and 95% CIs for cognitive-behavioral parameters in the visuospatial modality, in different intervention groups. The delta values are calculated as the second half of each block minus the first half of that block. The *P* values are computed by comparing the mean delta values with zero using the one-sample *t*-test. A significantly positive mean delta value indicates an increase in the parameter over the 8-minute course of the block.

Intervention	Parameter	Sex	*N*	Mean	SD	95% CI		Min	Max	*P*
Silence	Hit rate	Female	17	0.795	0.144	0.72	0.87	0.50	0.94	
		Male	14	0.852	0.140	0.77	0.93	0.47	1.00	
		Total	31	0.820	0.143	0.77	0.87	0.47	1.00	
	Delta hit rate	Female	17	-0.046	0.135	-0.12	0.02	-0.31	0.17	
		Male	14	-0.122	0.077	-0.17	-0.08	-0.26	0.00	
		Total	31	-0.080	0.117	-0.12	-0.04	-0.31	0.17	0.001
	FA rate	Female	17	0.081	0.072	0.04	0.12	0.01	0.27	
		Male	14	0.045	0.045	0.02	0.07	0.01	0.18	
		Total	31	0.065	0.063	0.04	0.09	0.01	0.27	
	Delta FA rate	Female	17	0.008	0.046	-0.02	0.03	-0.07	0.13	
		Male	14	-0.014	0.035	-0.03	0.01	-0.10	0.04	
		Total	31	-0.002	0.042	-0.02	0.01	-0.10	0.13	0.772
	*A*′	Female	17	0.913	0.073	0.88	0.95	0.69	0.98	
		Male	14	0.945	0.056	0.91	0.98	0.82	0.99	
		Total	31	0.927	0.067	0.90	0.95	0.69	0.99	
	Delta *A*′	Female	17	-0.019	0.051	-0.05	0.01	-0.12	0.06	
		Male	14	-0.028	0.029	-0.04	-0.01	-0.09	0.03	
		Total	31	-0.023	0.042	-0.04	-0.01	-0.12	0.06	0.005
	*B*′′	Female	17	0.391	0.326	0.22	0.56	-0.31	0.83	
		Male	14	0.402	0.483	0.12	0.68	-1.00	0.86	
		Total	31	0.396	0.397	0.25	0.54	-1.00	0.86	
	WM	Female	17	1.427	0.374	1.23	1.62	0.46	1.84	
		Male	14	1.613	0.340	1.42	1.81	0.79	1.91	
		Total	31	1.511	0.365	1.38	1.64	0.46	1.91	
	Delta WM	Female	17	-0.108	0.300	-0.26	0.05	-0.67	0.34	
		Male	14	-0.215	0.150	-0.30	-0.13	-0.46	-0.03	
		Total	31	-0.156	0.246	-0.25	-0.07	-0.67	0.34	0.001
	RT	Female	17	1.487	0.308	1.33	1.65	0.93	2.14	
		Male	14	1.439	0.191	1.33	1.55	1.17	1.72	
		Total	31	1.466	0.259	1.37	1.56	0.93	2.14	
	Delta RT	Female	17	0.025	0.213	-0.08	0.13	-0.35	0.46	
		Male	14	-0.048	0.176	-0.15	0.05	-0.36	0.32	
		Total	31	-0.008	0.197	-0.08	0.06	-0.36	0.46	0.819
	RTSD	Female	17	0.547	0.156	0.47	0.63	0.31	0.86	
		Male	14	0.521	0.131	0.45	0.60	0.33	0.79	
		Total	31	0.535	0.144	0.48	0.59	0.31	0.86	

Pure tone	Hit rate	Female	17	0.813	0.137	0.74	0.88	0.57	0.97	
		Male	14	0.850	0.109	0.79	0.91	0.65	1.00	
		Total	31	0.830	0.125	0.78	0.88	0.57	1.00	
	Delta hit rate	Female	17	-0.020	0.160	-0.10	0.06	-0.39	0.21	
		Male	14	-0.035	0.108	-0.10	0.03	-0.22	0.17	
		Total	31	-0.027	0.137	-0.08	0.02	-0.39	0.21	0.282
	FA rate	Female	17	0.097	0.110	0.04	0.15	0.01	0.47	
		Male	14	0.050	0.059	0.02	0.08	0.00	0.24	
		Total	31	0.076	0.092	0.04	0.11	0.00	0.47	
	Delta FA rate	Female	17	-0.016	0.047	-0.04	0.01	-0.12	0.08	
		Male	14	-0.022	0.028	-0.04	-0.01	-0.06	0.04	
		Total	31	-0.019	0.039	-0.03	0.00	-0.12	0.08	0.012
	*A*′	Female	17	0.912	0.086	0.87	0.96	0.62	0.98	
		Male	14	0.943	0.052	0.91	0.97	0.79	1.00	
		Total	31	0.926	0.073	0.90	0.95	0.62	1.00	
	Delta *A*′	Female	17	0.003	0.057	-0.03	0.03	-0.14	0.11	
		Male	14	-0.006	0.042	-0.03	0.02	-0.11	0.05	
		Total	31	-0.001	0.050	-0.02	0.02	-0.14	0.11	0.890
	*B*′′	Female	17	0.285	0.429	0.06	0.51	-0.58	0.91	
		Male	13	0.377	0.481	0.09	0.67	-1.00	0.80	
		Total	30	0.325	0.447	0.16	0.49	-1.00	0.91	
	WM	Female	17	1.431	0.394	1.23	1.63	0.26	1.81	
		Male	14	1.600	0.309	1.42	1.78	0.82	2.00	
		Total	31	1.508	0.363	1.37	1.64	0.26	2.00	
	Delta WM	Female	17	-0.008	0.323	-0.17	0.16	-0.81	0.46	
		Male	14	-0.027	0.240	-0.17	0.11	-0.50	0.38	
		Total	31	-0.017	0.284	-0.12	0.09	-0.81	0.46	0.746
	RT	Female	17	1.498	0.281	1.35	1.64	0.85	2.13	
		Male	14	1.483	0.214	1.36	1.61	0.98	1.82	
		Total	31	1.491	0.249	1.40	1.58	0.85	2.13	
	Delta RT	Female	17	-0.064	0.235	-0.18	0.06	-0.72	0.22	
		Male	14	-0.139	0.221	-0.27	-0.01	-0.64	0.29	
		Total	31	-0.098	0.228	-0.18	-0.01	-0.72	0.29	0.024
	RTSD	Female	17	0.554	0.126	0.49	0.62	0.29	0.81	
		Male	14	0.507	0.170	0.41	0.61	0.26	0.84	
		Total	31	0.533	0.147	0.48	0.59	0.26	0.84	

10 Hz BB	Hit rate	Female	17	0.817	0.143	0.74	0.89	0.42	0.97	
		Male	14	0.903	0.084	0.86	0.95	0.72	1.00	
		Total	31	0.856	0.126	0.81	0.90	0.42	1.00	
	Delta hit rate	Female	17	-0.008	0.113	-0.07	0.05	-0.20	0.25	
		Male	14	-0.008	0.077	-0.05	0.04	-0.13	0.13	
		Total	31	-0.008	0.097	-0.04	0.03	-0.20	0.25	0.637
	FA rate	Female	17	0.083	0.098	0.03	0.13	0.02	0.40	
		Male	14	0.053	0.045	0.03	0.08	0.01	0.15	
		Total	31	0.070	0.079	0.04	0.10	0.01	0.40	
	Delta FA rate	Female	17	-0.013	0.046	-0.04	0.01	-0.12	0.10	
		Male	14	-0.015	0.034	-0.03	0.01	-0.09	0.04	
		Total	31	-0.014	0.040	-0.03	0.00	-0.12	0.10	0.070
	*A*′	Female	17	0.918	0.084	0.87	0.96	0.64	0.99	
		Male	14	0.959	0.029	0.94	0.98	0.90	0.99	
		Total	31	0.937	0.067	0.91	0.96	0.64	0.99	
	Delta *A*′	Female	17	0.008	0.044	-0.01	0.03	-0.04	0.11	
		Male	14	0.002	0.023	-0.01	0.02	-0.03	0.04	
		Total	31	0.005	0.035	-0.01	0.02	-0.04	0.11	0.428
	*B*′′	Female	17	0.358	0.333	0.19	0.53	-0.16	0.83	
		Male	14	0.169	0.515	-0.13	0.47	-1.00	0.90	
		Total	31	0.273	0.428	0.12	0.43	-1.00	0.90	
	WM	Female	17	1.467	0.408	1.26	1.68	0.33	1.90	
		Male	14	1.701	0.202	1.58	1.82	1.28	1.93	
		Total	31	1.573	0.347	1.45	1.70	0.33	1.93	
	Delta WM	Female	17	0.009	0.239	-0.11	0.13	-0.34	0.52	
		Male	14	0.012	0.167	-0.08	0.11	-0.20	0.30	
		Total	31	0.011	0.206	-0.07	0.09	-0.34	0.52	0.777
	RT	Female	17	1.429	0.232	1.31	1.55	1.02	1.95	
		Male	14	1.456	0.207	1.34	1.58	1.05	1.78	
		Total	31	1.441	0.218	1.36	1.52	1.02	1.95	
	Delta RT	Female	17	-0.060	0.213	-0.17	0.05	-0.52	0.22	
		Male	14	-0.058	0.164	-0.15	0.04	-0.41	0.24	
		Total	31	-0.059	0.189	-0.13	0.01	-0.52	0.24	0.093
	RTSD	Female	17	0.518	0.113	0.46	0.58	0.29	0.75	
		Male	14	0.496	0.128	0.42	0.57	0.33	0.69	
		Total	31	0.508	0.118	0.46	0.55	0.29	0.75	

16 Hz BB	Hit rate	Female	17	0.827	0.177	0.74	0.92	0.30	1.00	
		Male	14	0.855	0.103	0.80	0.91	0.57	0.97	
		Total	31	0.840	0.147	0.79	0.89	0.30	1.00	
	Delta hit rate	Female	17	-0.096	0.130	-0.16	-0.03	-0.29	0.19	
		Male	14	-0.047	0.169	-0.14	0.05	-0.37	0.25	
		Total	31	-0.074	0.149	-0.13	-0.02	-0.37	0.25	0.009
	FA rate	Female	17	0.093	0.108	0.04	0.15	0.00	0.39	
		Male	14	0.046	0.043	0.02	0.07	0.00	0.12	
		Total	31	0.072	0.087	0.04	0.10	0.00	0.39	
	Delta FA rate	Female	17	-0.026	0.065	-0.06	0.01	-0.15	0.05	
		Male	14	0.007	0.039	-0.01	0.03	-0.04	0.11	
		Total	31	-0.011	0.057	-0.03	0.01	-0.15	0.11	0.291
	*A*′	Female	17	0.918	0.088	0.87	0.96	0.64	1.00	
		Male	14	0.948	0.034	0.93	0.97	0.85	0.99	
		Total	31	0.932	0.069	0.91	0.96	0.64	1.00	
	Delta *A*′	Female	17	-0.025	0.048	-0.05	0.00	-0.16	0.04	
		Male	14	-0.015	0.043	-0.04	0.01	-0.09	0.06	
		Total	31	-0.020	0.045	-0.04	0.00	-0.16	0.06	0.018
	*B*′′	Female	16	0.266	0.393	0.06	0.48	-0.69	0.83	
		Male	14	0.494	0.459	0.23	0.76	-0.42	1.00	
		Total	30	0.372	0.433	0.21	0.53	-0.69	1.00	
	WM	Female	17	1.469	0.454	1.24	1.70	0.32	2.00	
		Male	14	1.617	0.225	1.49	1.75	0.99	1.93	
		Total	31	1.536	0.371	1.40	1.67	0.32	2.00	
	Delta WM	Female	17	-0.140	0.269	-0.28	0.00	-0.66	0.34	
		Male	14	-0.109	0.329	-0.30	0.08	-0.73	0.46	
		Total	31	-0.126	0.292	-0.23	-0.02	-0.73	0.46	0.023
	RT	Female	17	1.541	0.273	1.40	1.68	0.90	2.05	
		Male	14	1.481	0.243	1.34	1.62	1.11	1.84	
		Total	31	1.514	0.257	1.42	1.61	0.90	2.05	
	Delta RT	Female	17	-0.041	0.184	-0.14	0.05	-0.43	0.27	
		Male	14	0.030	0.194	-0.08	0.14	-0.21	0.31	
		Total	31	-0.009	0.189	-0.08	0.06	-0.43	0.31	0.795
	RTSD	Female	17	0.555	0.137	0.48	0.63	0.33	0.83	
		Male	14	0.506	0.079	0.46	0.55	0.38	0.62	
		Total	31	0.533	0.116	0.49	0.58	0.33	0.83	

40 Hz BB	Hit rate	Female	17	0.812	0.174	0.72	0.90	0.38	1.00	
		Male	14	0.851	0.067	0.81	0.89	0.73	0.93	
		Total	31	0.830	0.136	0.78	0.88	0.38	1.00	
	Delta hit rate	Female	17	-0.076	0.156	-0.16	0.00	-0.53	0.12	
		Male	14	0.031	0.147	-0.05	0.12	-0.10	0.44	
		Total	31	-0.027	0.159	-0.09	0.03	-0.53	0.44	0.345
	FA rate	Female	17	0.074	0.078	0.03	0.11	0.01	0.32	
		Male	14	0.050	0.058	0.02	0.08	0.00	0.20	
		Total	31	0.064	0.070	0.04	0.09	0.00	0.32	
	Delta FA rate	Female	17	-0.016	0.052	-0.04	0.01	-0.13	0.10	
		Male	14	-0.004	0.021	-0.02	0.01	-0.05	0.03	
		Total	31	-0.010	0.041	-0.03	0.00	-0.13	0.10	0.162
	*A*′	Female	17	0.917	0.095	0.87	0.97	0.61	1.00	
		Male	14	0.944	0.037	0.92	0.97	0.85	0.98	
		Total	31	0.929	0.075	0.90	0.96	0.61	1.00	
	Delta *A*′	Female	17	-0.032	0.097	-0.08	0.02	-0.39	0.05	
		Male	14	0.014	0.061	-0.02	0.05	-0.03	0.21	
		Total	31	-0.011	0.085	-0.04	0.02	-0.39	0.21	0.457
	*B*′′	Female	17	0.246	0.539	-0.03	0.52	-1.00	0.86	
		Male	14	0.559	0.312	0.38	0.74	0.10	1.00	
		Total	31	0.388	0.471	0.21	0.56	-1.00	1.00	
	WM	Female	17	1.475	0.449	1.24	1.71	0.24	1.97	
		Male	14	1.601	0.228	1.47	1.73	1.07	1.87	
		Total	31	1.532	0.366	1.40	1.67	0.24	1.97	
	Delta WM	Female	17	-0.119	0.254	-0.25	0.01	-0.79	0.24	
		Male	14	0.070	0.318	-0.11	0.25	-0.22	0.97	
		Total	31	-0.034	0.296	-0.14	0.07	-0.79	0.97	0.530
	RT	Female	17	1.463	0.255	1.33	1.59	0.90	1.97	
		Male	14	1.519	0.224	1.39	1.65	1.13	1.93	
		Total	31	1.488	0.239	1.40	1.58	0.90	1.97	
	Delta RT	Female	17	-0.130	0.238	-0.25	-0.01	-0.56	0.17	
		Male	14	-0.067	0.244	-0.21	0.07	-0.46	0.36	
		Total	31	-0.101	0.239	-0.19	-0.01	-0.56	0.36	0.025
	RTSD	Female	17	0.528	0.145	0.45	0.60	0.22	0.81	
		Male	14	0.525	0.108	0.46	0.59	0.37	0.70	
		Total	31	0.527	0.127	0.48	0.57	0.22	0.81	

BB: binaural beat; FA rate: false alarm rate; *A*′: sensitivity; *B*^″^: response bias; WM: working memory; RT: response time; RTSD: response time standard deviation; SD: standard deviation; CI: confidence interval; Min: minimum; Max: maximum.

**Table 2:** Descriptive statistics and 95% CIs for cognitive-behavioral parameters in the auditory-verbal modality, in different intervention groups. The delta values are calculated as the second half of each block minus the first half of that block. The *P* values are calculated by comparing the mean delta values with zero, using the one-sample *t*-test. A significantly negative mean delta value shows a decline in the parameter in 8 minutes.

Intervention	Parameter	Sex	*N*	Mean	SD	95% CI		Min	Max	*P*
Silence	Hit rate	Female	17	0.865	0.098	0.81	0.92	0.67	0.97	
		Male	14	0.913	0.098	0.86	0.97	0.67	1.00	
		Total	31	0.887	0.099	0.85	0.92	0.67	1.00	
	Delta hit rate	Female	17	0.002	0.115	-0.06	0.06	-0.26	0.17	
		Male	14	0.004	0.115	-0.06	0.07	-0.35	0.14	
		Total	31	0.003	0.113	-0.04	0.04	-0.35	0.17	0.898
	FA rate	Female	17	0.126	0.078	0.09	0.17	0.03	0.34	
		Male	14	0.090	0.063	0.05	0.13	0.02	0.28	
		Total	31	0.110	0.073	0.08	0.14	0.02	0.34	
	Delta FA rate	Female	17	0.015	0.051	-0.01	0.04	-0.07	0.13	
		Male	14	0.018	0.062	-0.02	0.05	-0.09	0.15	
		Total	31	0.016	0.055	0.00	0.04	-0.09	0.15	0.107
	*A*′	Female	17	0.923	0.052	0.90	0.95	0.75	0.98	
		Male	14	0.951	0.035	0.93	0.97	0.88	1.00	
		Total	31	0.936	0.047	0.92	0.95	0.75	1.00	
	Delta *A*′	Female	17	-0.006	0.047	-0.03	0.02	-0.12	0.09	
		Male	14	-0.004	0.042	-0.03	0.02	-0.13	0.07	
		Total	31	-0.005	0.044	-0.02	0.01	-0.13	0.09	0.536
	*B*′′	Female	17	-0.027	0.440	-0.25	0.20	-0.67	0.59	
		Male	14	-0.284	0.609	-0.64	0.07	-1.00	0.57	
		Total	31	-0.143	0.530	-0.34	0.05	-1.00	0.59	
	WM	Female	17	1.479	0.269	1.34	1.62	0.66	1.88	
		Male	14	1.645	0.235	1.51	1.78	1.18	1.97	
		Total	31	1.554	0.264	1.46	1.65	0.66	1.97	
	Delta WM	Female	17	-0.027	0.276	-0.17	0.11	-0.68	0.47	
		Male	14	-0.028	0.276	-0.19	0.13	-0.82	0.45	
		Total	31	-0.028	0.271	-0.13	0.07	-0.82	0.47	0.575
	RT	Female	17	1.551	0.229	1.43	1.67	1.26	2.03	
		Male	14	1.576	0.186	1.47	1.68	1.31	2.00	
		Total	31	1.563	0.208	1.49	1.64	1.26	2.03	
	Delta RT	Female	17	-0.021	0.194	-0.12	0.08	-0.41	0.36	
		Male	14	-0.045	0.192	-0.16	0.07	-0.50	0.23	
		Total	31	-0.032	0.190	-0.10	0.04	-0.50	0.36	0.357
	RTSD	Female	17	0.474	0.130	0.41	0.54	0.29	0.70	
		Male	14	0.473	0.092	0.42	0.53	0.24	0.60	
		Total	31	0.473	0.113	0.43	0.51	0.24	0.70	

Pure tone	Hit rate	Female	17	0.868	0.080	0.83	0.91	0.70	0.97	
		Male	14	0.888	0.118	0.82	0.96	0.53	1.00	
		Total	31	0.877	0.098	0.84	0.91	0.53	1.00	
	Delta hit rate	Female	17	0.037	0.166	-0.05	0.12	-0.25	0.40	
		Male	14	-0.045	0.140	-0.13	0.04	-0.27	0.26	
		Total	31	0.000	0.158	-0.06	0.06	-0.27	0.40	0.999
	FA rate	Female	17	0.140	0.143	0.07	0.21	0.03	0.64	
		Male	14	0.091	0.058	0.06	0.12	0.02	0.23	
		Total	31	0.118	0.114	0.08	0.16	0.02	0.64	
	Delta FA rate	Female	17	0.032	0.054	0.00	0.06	-0.09	0.09	
		Male	14	0.028	0.038	0.01	0.05	-0.04	0.10	
		Total	31	0.031	0.047	0.01	0.05	-0.09	0.10	0.001
	*A*′	Female	17	0.922	0.048	0.90	0.95	0.76	0.98	
		Male	14	0.943	0.041	0.92	0.97	0.85	1.00	
		Total	31	0.931	0.046	0.91	0.95	0.76	1.00	
	Delta *A*′	Female	17	0.004	0.055	-0.02	0.03	-0.10	0.11	
		Male	14	-0.021	0.050	-0.05	0.01	-0.09	0.10	
		Total	31	-0.007	0.053	-0.03	0.01	-0.10	0.11	0.441
	*B*′′	Female	17	0.036	0.411	-0.18	0.25	-0.70	0.68	
		Male	14	-0.065	0.436	-0.32	0.19	-1.00	0.67	
		Total	31	-0.010	0.419	-0.16	0.14	-1.00	0.68	
	WM	Female	17	1.455	0.283	1.31	1.60	0.53	1.81	
		Male	14	1.594	0.267	1.44	1.75	0.96	1.97	
		Total	31	1.518	0.280	1.42	1.62	0.53	1.97	
	Delta WM	Female	17	0.009	0.361	-0.18	0.19	-0.64	0.80	
		Male	14	-0.146	0.309	-0.32	0.03	-0.63	0.59	
		Total	31	-0.061	0.342	-0.19	0.06	-0.64	0.80	0.328
	RT	Female	17	1.512	0.226	1.40	1.63	1.04	1.90	
		Male	14	1.588	0.203	1.47	1.71	1.32	1.97	
		Total	31	1.546	0.216	1.47	1.63	1.04	1.97	
	Delta RT	Female	17	-0.090	0.131	-0.16	-0.02	-0.32	0.13	
		Male	14	0.019	0.150	-0.07	0.11	-0.26	0.22	
		Total	31	-0.041	0.148	-0.09	0.01	-0.32	0.22	0.136
	RTSD	Female	17	0.456	0.149	0.38	0.53	0.23	0.69	
		Male	14	0.465	0.080	0.42	0.51	0.37	0.65	
		Total	31	0.460	0.121	0.42	0.50	0.23	0.69	

10 Hz BB	Hit rate	Female	17	0.846	0.149	0.77	0.92	0.37	1.00	
		Male	14	0.870	0.114	0.80	0.94	0.65	1.00	
		Total	31	0.857	0.133	0.81	0.91	0.37	1.00	
	Delta hit rate	Female	17	-0.024	0.160	-0.11	0.06	-0.30	0.30	
		Male	14	-0.019	0.125	-0.09	0.05	-0.17	0.28	
		Total	31	-0.022	0.143	-0.07	0.03	-0.30	0.30	0.408
	FA rate	Female	17	0.136	0.124	0.07	0.20	0.04	0.57	
		Male	14	0.083	0.038	0.06	0.10	0.02	0.16	
		Total	31	0.112	0.098	0.08	0.15	0.02	0.57	
	Delta FA rate	Female	17	0.008	0.058	-0.02	0.04	-0.10	0.11	
		Male	14	0.011	0.048	-0.02	0.04	-0.07	0.09	
		Total	31	0.010	0.053	-0.01	0.03	-0.10	0.11	0.317
	*A*′	Female	17	0.914	0.066	0.88	0.95	0.71	0.99	
		Male	14	0.941	0.034	0.92	0.96	0.88	0.98	
		Total	31	0.926	0.055	0.91	0.95	0.71	0.99	
	Delta *A*′	Female	17	-0.009	0.058	-0.04	0.02	-0.11	0.07	
		Male	14	-0.009	0.038	-0.03	0.01	-0.05	0.06	
		Total	31	-0.009	0.049	-0.03	0.01	-0.11	0.07	0.319
	*B*′′	Female	17	-0.056	0.479	-0.30	0.19	-1.00	0.70	
		Male	14	-0.020	0.567	-0.35	0.31	-1.00	0.84	
		Total	31	-0.040	0.512	-0.23	0.15	-1.00	0.84	
	WM	Female	17	1.419	0.363	1.23	1.61	0.47	1.91	
		Male	14	1.575	0.228	1.44	1.71	1.19	1.88	
		Total	31	1.489	0.315	1.37	1.60	0.47	1.91	
	Delta WM	Female	17	-0.064	0.365	-0.25	0.12	-0.66	0.51	
		Male	14	-0.061	0.256	-0.21	0.09	-0.36	0.44	
		Total	31	-0.062	0.316	-0.18	0.05	-0.66	0.51	0.280
	RT	Female	17	1.541	0.232	1.42	1.66	1.12	1.92	
		Male	14	1.610	0.224	1.48	1.74	1.29	2.04	
		Total	31	1.572	0.227	1.49	1.66	1.12	2.04	
	Delta RT	Female	17	0.023	0.211	-0.09	0.13	-0.49	0.27	
		Male	14	-0.043	0.235	-0.18	0.09	-0.52	0.31	
		Total	31	-0.007	0.221	-0.09	0.07	-0.52	0.31	0.862
	RTSD	Female	17	0.456	0.105	0.40	0.51	0.24	0.69	
		Male	14	0.488	0.123	0.42	0.56	0.31	0.74	
		Total	31	0.470	0.113	0.43	0.51	0.24	0.74	

16 Hz BB	Hit rate	Female	17	0.854	0.114	0.80	0.91	0.60	1.00	
		Male	14	0.905	0.106	0.84	0.97	0.67	1.00	
		Total	31	0.877	0.112	0.84	0.92	0.60	1.00	
	Delta hit rate	Female	17	-0.083	0.085	-0.13	-0.04	-0.25	0.11	
		Male	14	-0.024	0.099	-0.08	0.03	-0.23	0.11	
		Total	31	-0.056	0.095	-0.09	-0.02	-0.25	0.11	0.003
	FA rate	Female	17	0.139	0.118	0.08	0.20	0.04	0.49	
		Male	14	0.084	0.040	0.06	0.11	0.00	0.16	
		Total	31	0.114	0.094	0.08	0.15	0.00	0.49	
	Delta FA rate	Female	17	0.014	0.066	-0.02	0.05	-0.11	0.11	
		Male	14	0.037	0.045	0.01	0.06	-0.03	0.15	
		Total	31	0.025	0.058	0.00	0.05	-0.11	0.15	0.023
	*A*′	Female	17	0.915	0.061	0.88	0.95	0.73	0.98	
		Male	14	0.951	0.029	0.93	0.97	0.88	0.99	
		Total	31	0.931	0.052	0.91	0.95	0.73	0.99	
	Delta *A*′	Female	17	-0.035	0.039	-0.05	-0.01	-0.14	0.02	
		Male	14	-0.018	0.035	-0.04	0.00	-0.08	0.04	
		Total	31	-0.027	0.038	-0.04	-0.01	-0.14	0.04	<0.0005
	*B*′′	Female	17	0.007	0.418	-0.21	0.22	-1.00	0.70	
		Male	14	-0.126	0.667	-0.51	0.26	-1.00	1.00	
		Total	31	-0.053	0.539	-0.25	0.14	-1.00	1.00	
	WM	Female	17	1.430	0.327	1.26	1.60	0.56	1.81	
		Male	14	1.642	0.199	1.53	1.76	1.19	1.93	
		Total	31	1.526	0.293	1.42	1.63	0.56	1.93	
	Delta WM	Female	17	-0.194	0.177	-0.28	-0.10	-0.50	0.11	
		Male	14	-0.123	0.233	-0.26	0.01	-0.54	0.29	
		Total	31	-0.162	0.204	-0.24	-0.09	-0.54	0.29	<0.0005
	RT	Female	17	1.526	0.232	1.41	1.65	1.09	1.92	
		Male	14	1.587	0.214	1.46	1.71	1.16	2.02	
		Total	31	1.554	0.223	1.47	1.64	1.09	2.02	
	Delta RT	Female	17	-0.033	0.166	-0.12	0.05	-0.44	0.28	
		Male	14	-0.087	0.204	-0.20	0.03	-0.60	0.11	
		Total	31	-0.057	0.183	-0.12	0.01	-0.60	0.28	0.092
	RTSD	Female	17	0.461	0.130	0.39	0.53	0.25	0.69	
		Male	14	0.461	0.076	0.42	0.51	0.29	0.57	
		Total	31	0.461	0.108	0.42	0.50	0.25	0.69	

40 Hz BB	Hit rate	Female	17	0.877	0.109	0.82	0.93	0.63	1.00	
		Male	14	0.915	0.093	0.86	0.97	0.73	1.00	
		Total	31	0.894	0.102	0.86	0.93	0.63	1.00	
	Delta hit rate	Female	17	-0.023	0.125	-0.09	0.04	-0.28	0.21	
		Male	14	-0.062	0.098	-0.12	-0.01	-0.25	0.08	
		Total	31	-0.041	0.113	-0.08	0.00	-0.28	0.21	0.054
	FA rate	Female	17	0.132	0.087	0.09	0.18	0.03	0.40	
		Male	14	0.096	0.057	0.06	0.13	0.03	0.23	
		Total	31	0.116	0.076	0.09	0.14	0.03	0.40	
	Delta FA rate	Female	17	0.014	0.057	-0.02	0.04	-0.06	0.14	
		Male	14	0.009	0.049	-0.02	0.04	-0.05	0.10	
		Total	31	0.012	0.053	-0.01	0.03	-0.06	0.14	0.220
	*A*′	Female	17	0.925	0.052	0.90	0.95	0.81	0.99	
		Male	14	0.950	0.034	0.93	0.97	0.88	0.99	
		Total	31	0.936	0.046	0.92	0.95	0.81	0.99	
	Delta *A*′	Female	17	-0.013	0.056	-0.04	0.02	-0.11	0.09	
		Male	14	-0.023	0.046	-0.05	0.00	-0.13	0.03	
		Total	31	-0.017	0.051	-0.04	0.00	-0.13	0.09	0.068
	*B*′′	Female	17	-0.183	0.495	-0.44	0.07	-1.00	0.43	
		Male	14	-0.258	0.621	-0.62	0.10	-1.00	0.71	
		Total	31	-0.217	0.547	-0.42	-0.02	-1.00	0.71	
	WM	Female	17	1.490	0.311	1.33	1.65	0.87	1.91	
		Male	14	1.639	0.218	1.51	1.76	1.21	1.90	
		Total	31	1.557	0.279	1.46	1.66	0.87	1.91	
	Delta WM	Female	17	-0.074	0.312	-0.23	0.09	-0.66	0.47	
		Male	14	-0.143	0.266	-0.30	0.01	-0.67	0.19	
		Total	31	-0.105	0.290	-0.21	0.00	-0.67	0.47	0.052
	RT	Female	17	1.534	0.217	1.42	1.65	1.21	1.90	
		Male	14	1.530	0.198	1.42	1.64	1.19	1.97	
		Total	31	1.532	0.205	1.46	1.61	1.19	1.97	
	Delta RT	Female	17	-0.089	0.201	-0.19	0.01	-0.56	0.28	
		Male	14	-0.021	0.130	-0.10	0.05	-0.20	0.27	
		Total	31	-0.058	0.173	-0.12	0.01	-0.56	0.28	0.072
	RTSD	Female	17	0.493	0.124	0.43	0.56	0.30	0.70	
		Male	14	0.430	0.100	0.37	0.49	0.19	0.55	
		Total	31	0.465	0.116	0.42	0.51	0.19	0.70	

BB: binaural beat; FA rate: false alarm rate; *A*′: sensitivity; *B*^″^: response bias; WM: working memory; RT: response time; RTSD: response time standard deviation; SD: standard deviation; CI: confidence interval; Min: minimum; Max: maximum.

**Table 3:** Descriptive statistics and 95% CIs for cognitive-behavioral parameters in the visuospatial modality, in different time-blocks. The delta values are computed as the second half of each block minus the first half of that block. The *P* values are calculated by comparing the mean delta values with zero, using the one-sample t-test. A significantly positive mean delta value indicates an increase in the parameter over the 8-minute time of the block.

Time-block	Parameter	Sex	N	Mean	SD	95% CI		Min	Max	*P*
1	Hit Rate	Female	17	0.782	0.166	0.70	0.87	0.38	0.97	
		Male	14	0.833	0.096	0.78	0.89	0.63	0.97	
		Total	31	0.805	0.139	0.75	0.86	0.38	0.97	
	Delta Hit Rate	Female	17	-0.068	0.176	-0.16	0.02	-0.53	0.15	
		Male	14	-0.059	0.133	-0.14	0.02	-0.37	0.14	
		Total	31	-0.064	0.156	-0.12	-0.01	-0.53	0.15	0.029
	FA Rate	Female	17	0.090	0.092	0.04	0.14	0.01	0.32	
		Male	14	0.070	0.051	0.04	0.10	0.00	0.18	
		Total	31	0.081	0.076	0.05	0.11	0.00	0.32	
	Delta FA Rate	Female	17	-0.010	0.049	-0.04	0.01	-0.13	0.05	
		Male	14	0.002	0.039	-0.02	0.02	-0.06	0.11	
		Total	31	-0.005	0.044	-0.02	0.01	-0.13	0.11	0.536
	A'	Female	17	0.905	0.090	0.86	0.95	0.61	0.98	
		Male	14	0.932	0.043	0.91	0.96	0.82	0.98	
		Total	31	0.917	0.073	0.89	0.94	0.61	0.98	
	Delta A'	Female	17	-0.033	0.103	-0.09	0.02	-0.39	0.07	
		Male	14	-0.020	0.038	-0.04	0.00	-0.09	0.04	
		Total	31	-0.027	0.080	-0.06	0.00	-0.39	0.07	0.066
	B''	Female	17	0.346	0.434	0.12	0.57	-0.58	0.91	
		Male	14	0.359	0.390	0.13	0.58	-0.42	1.00	
		Total	31	0.352	0.408	0.20	0.50	-0.58	1.00	
	WM	Female	17	1.386	0.410	1.17	1.60	0.24	1.84	
		Male	14	1.527	0.250	1.38	1.67	0.90	1.82	
		Total	31	1.450	0.349	1.32	1.58	0.24	1.84	
	Delta WM	Female	17	-0.115	0.337	-0.29	0.06	-0.79	0.46	
		Male	14	-0.122	0.254	-0.27	0.02	-0.73	0.32	
		Total	31	-0.118	0.298	-0.23	-0.01	-0.79	0.46	0.034
	RT	Female	17	1.551	0.263	1.42	1.69	1.05	2.10	
		Male	14	1.582	0.206	1.46	1.70	1.13	1.84	
		Total	31	1.565	0.236	1.48	1.65	1.05	2.10	
	Delta RT	Female	17	-0.020	0.206	-0.13	0.09	-0.56	0.46	
		Male	14	-0.023	0.168	-0.12	0.07	-0.35	0.31	
		Total	31	-0.021	0.187	-0.09	0.05	-0.56	0.46	0.534
	RTSD	Female	17	0.555	0.131	0.49	0.62	0.31	0.81	
		Male	14	0.530	0.125	0.46	0.60	0.33	0.70	
		Total	31	0.544	0.127	0.50	0.59	0.31	0.81	

2	Hit Rate	Female	17	0.787	0.135	0.72	0.86	0.50	0.93	
		Male	14	0.856	0.075	0.81	0.90	0.73	0.97	
		Total	31	0.818	0.116	0.78	0.86	0.50	0.97	
	Delta Hit Rate	Female	17	-0.015	0.108	-0.07	0.04	-0.21	0.17	
		Male	14	0.010	0.135	-0.07	0.09	-0.12	0.44	
		Total	31	-0.004	0.119	-0.05	0.04	-0.21	0.44	0.850
	FA Rate	Female	17	0.095	0.080	0.05	0.14	0.02	0.27	
		Male	14	0.054	0.051	0.02	0.08	0.01	0.20	
		Total	31	0.077	0.071	0.05	0.10	0.01	0.27	
	Delta FA Rate	Female	17	-0.038	0.045	-0.06	-0.01	-0.12	0.03	
		Male	14	-0.030	0.032	-0.05	-0.01	-0.09	0.03	
		Total	31	-0.034	0.039	-0.05	-0.02	-0.12	0.03	<0.0005
	A'	Female	17	0.905	0.072	0.87	0.94	0.69	0.98	
		Male	14	0.945	0.035	0.92	0.97	0.85	0.99	
		Total	31	0.923	0.061	0.90	0.95	0.69	0.99	
	Delta A'	Female	17	0.007	0.031	-0.01	0.02	-0.07	0.06	
		Male	14	0.018	0.059	-0.02	0.05	-0.03	0.21	
		Total	31	0.012	0.045	-0.01	0.03	-0.07	0.21	0.165
	B''	Female	17	0.371	0.306	0.21	0.53	-0.25	0.74	
		Male	14	0.419	0.304	0.24	0.60	-0.15	0.86	
		Total	31	0.393	0.301	0.28	0.50	-0.25	0.86	
	WM	Female	17	1.384	0.369	1.19	1.57	0.46	1.81	
		Male	14	1.604	0.215	1.48	1.73	1.07	1.90	
		Total	31	1.483	0.324	1.36	1.60	0.46	1.90	
	Delta WM	Female	17	0.045	0.174	-0.04	0.13	-0.24	0.34	
		Male	14	0.079	0.299	-0.09	0.25	-0.22	0.97	
		Total	31	0.060	0.235	-0.03	0.15	-0.24	0.97	0.164
	RT	Female	17	1.536	0.271	1.40	1.68	0.93	2.14	
		Male	14	1.532	0.173	1.43	1.63	1.17	1.82	
		Total	31	1.534	0.228	1.45	1.62	0.93	2.14	
	Delta RT	Female	17	-0.079	0.199	-0.18	0.02	-0.49	0.27	
		Male	14	-0.096	0.253	-0.24	0.05	-0.64	0.36	
		Total	31	-0.087	0.221	-0.17	-0.01	-0.64	0.36	0.037
	RTSD	Female	17	0.572	0.154	0.49	0.65	0.32	0.86	
		Male	14	0.517	0.110	0.45	0.58	0.33	0.67	
		Total	31	0.547	0.137	0.50	0.60	0.32	0.86	

3	Hit Rate	Female	17	0.810	0.161	0.73	0.89	0.42	0.94	
		Male	14	0.844	0.137	0.76	0.92	0.47	1.00	
		Total	31	0.825	0.149	0.77	0.88	0.42	1.00	
	Delta Hit Rate	Female	17	-0.103	0.159	-0.18	-0.02	-0.39	0.15	
		Male	14	-0.063	0.108	-0.13	0.00	-0.22	0.17	
		Total	31	-0.085	0.137	-0.14	-0.03	-0.39	0.17	0.002
	FA Rate	Female	17	0.088	0.094	0.04	0.14	0.01	0.39	
		Male	14	0.048	0.060	0.01	0.08	0.00	0.24	
		Total	31	0.070	0.082	0.04	0.10	0.00	0.39	
	Delta FA Rate	Female	17	-0.001	0.059	-0.03	0.03	-0.15	0.13	
		Male	14	-0.009	0.034	-0.03	0.01	-0.10	0.04	
		Total	31	-0.005	0.049	-0.02	0.01	-0.15	0.13	0.605
	A'	Female	17	0.914	0.085	0.87	0.96	0.64	0.98	
		Male	14	0.941	0.060	0.91	0.98	0.79	0.99	
		Total	31	0.926	0.075	0.90	0.95	0.64	0.99	
	Delta A'	Female	17	-0.030	0.055	-0.06	0.00	-0.14	0.06	
		Male	14	-0.015	0.037	-0.04	0.01	-0.11	0.05	
		Total	31	-0.023	0.048	-0.04	-0.01	-0.14	0.06	0.011
	B''	Female	17	0.314	0.349	0.13	0.49	-0.41	0.86	
		Male	14	0.471	0.495	0.19	0.76	-1.00	1.00	
		Total	31	0.385	0.421	0.23	0.54	-1.00	1.00	
	WM	Female	17	1.445	0.422	1.23	1.66	0.32	1.82	
		Male	14	1.591	0.355	1.39	1.80	0.79	1.93	
		Total	31	1.511	0.394	1.37	1.66	0.32	1.93	
	Delta WM	Female	17	-0.203	0.334	-0.37	-0.03	-0.81	0.32	
		Male	14	-0.108	0.205	-0.23	0.01	-0.45	0.38	
		Total	31	-0.160	0.283	-0.26	-0.06	-0.81	0.38	0.004
	RT	Female	17	1.484	0.279	1.34	1.63	0.90	2.05	
		Male	14	1.463	0.199	1.35	1.58	1.11	1.72	
		Total	31	1.474	0.243	1.39	1.56	0.90	2.05	
	Delta RT	Female	17	-0.052	0.156	-0.13	0.03	-0.37	0.21	
		Male	14	-0.078	0.212	-0.20	0.04	-0.41	0.30	
		Total	31	-0.064	0.181	-0.13	0.00	-0.41	0.30	0.059
	RTSD	Female	17	0.534	0.146	0.46	0.61	0.22	0.78	
		Male	14	0.521	0.138	0.44	0.60	0.33	0.79	
		Total	31	0.528	0.140	0.48	0.58	0.22	0.79	

4	Hit Rate	Female	17	0.849	0.170	0.76	0.94	0.30	1.00	
		Male	14	0.892	0.086	0.84	0.94	0.74	1.00	
		Total	31	0.869	0.138	0.82	0.92	0.30	1.00	
	Delta Hit Rate	Female	17	-0.020	0.125	-0.08	0.04	-0.29	0.21	
		Male	14	0.009	0.120	-0.06	0.08	-0.21	0.25	
		Total	31	-0.007	0.122	-0.05	0.04	-0.29	0.25	0.765
	FA Rate	Female	17	0.079	0.113	0.02	0.14	0.00	0.47	
		Male	14	0.035	0.036	0.01	0.06	0.00	0.12	
		Total	31	0.059	0.089	0.03	0.09	0.00	0.47	
	Delta FA Rate	Female	17	0.009	0.058	-0.02	0.04	-0.13	0.10	
		Male	14	0.002	0.025	-0.01	0.02	-0.04	0.04	
		Total	31	0.006	0.046	-0.01	0.02	-0.13	0.10	0.453
	A'	Female	17	0.929	0.093	0.88	0.98	0.62	1.00	
		Male	14	0.962	0.028	0.95	0.98	0.91	1.00	
		Total	31	0.944	0.072	0.92	0.97	0.62	1.00	
	Delta A'	Female	17	-0.009	0.052	-0.04	0.02	-0.16	0.11	
		Male	14	0.000	0.035	-0.02	0.02	-0.08	0.06	
		Total	31	-0.005	0.044	-0.02	0.01	-0.16	0.11	0.541
	B''	Female	16	0.298	0.400	0.08	0.51	-0.69	0.83	
		Male	13	0.371	0.535	0.05	0.69	-1.00	0.90	
		Total	29	0.331	0.458	0.16	0.50	-1.00	0.90	
	WM	Female	17	1.541	0.458	1.31	1.78	0.26	2.00	
		Male	14	1.715	0.201	1.60	1.83	1.34	2.00	
		Total	31	1.619	0.370	1.48	1.76	0.26	2.00	
	Delta WM	Female	17	-0.058	0.225	-0.17	0.06	-0.66	0.34	
		Male	14	0.013	0.247	-0.13	0.16	-0.50	0.46	
		Total	31	-0.026	0.234	-0.11	0.06	-0.66	0.46	0.546
	RT	Female	17	1.448	0.264	1.31	1.58	0.90	1.93	
		Male	14	1.402	0.210	1.28	1.52	0.98	1.78	
		Total	31	1.427	0.238	1.34	1.51	0.90	1.93	
	Delta RT	Female	17	-0.057	0.244	-0.18	0.07	-0.53	0.21	
		Male	14	-0.039	0.204	-0.16	0.08	-0.43	0.32	
		Total	31	-0.049	0.223	-0.13	0.03	-0.53	0.32	0.233
	RTSD	Female	17	0.514	0.114	0.45	0.57	0.29	0.71	
		Male	14	0.475	0.155	0.39	0.56	0.26	0.84	
		Total	31	0.496	0.133	0.45	0.55	0.26	0.84	

5	Hit Rate	Female	17	0.834	0.135	0.76	0.90	0.57	1.00	
		Male	14	0.886	0.110	0.82	0.95	0.57	1.00	
		Total	31	0.857	0.125	0.81	0.90	0.57	1.00	
	Delta Hit Rate	Female	17	-0.041	0.121	-0.10	0.02	-0.22	0.25	
		Male	14	-0.078	0.133	-0.15	0.00	-0.33	0.15	
		Total	31	-0.058	0.126	-0.10	-0.01	-0.33	0.25	0.016
	FA Rate	Female	17	0.077	0.091	0.03	0.12	0.02	0.40	
		Male	14	0.038	0.042	0.01	0.06	0.00	0.15	
		Total	31	0.060	0.075	0.03	0.09	0.00	0.40	
	Delta FA Rate	Female	17	-0.024	0.037	-0.04	0.00	-0.12	0.04	
		Male	14	-0.012	0.025	-0.03	0.00	-0.06	0.04	
		Total	31	-0.018	0.032	-0.03	-0.01	-0.12	0.04	0.003
	A'	Female	17	0.925	0.082	0.88	0.97	0.64	1.00	
		Male	14	0.959	0.037	0.94	0.98	0.85	1.00	
		Total	31	0.940	0.067	0.92	0.96	0.64	1.00	
	Delta A'	Female	17	0.000	0.046	-0.02	0.02	-0.05	0.11	
		Male	14	-0.017	0.036	-0.04	0.00	-0.08	0.04	
		Total	31	-0.007	0.042	-0.02	0.01	-0.08	0.11	0.334
	B''	Female	17	0.218	0.532	-0.06	0.49	-1.00	0.76	
		Male	14	0.380	0.593	0.04	0.72	-1.00	1.00	
		Total	31	0.291	0.557	0.09	0.50	-1.00	1.00	
	WM	Female	17	1.514	0.396	1.31	1.72	0.33	1.97	
		Male	14	1.695	0.247	1.55	1.84	0.99	1.97	
		Total	31	1.596	0.344	1.47	1.72	0.33	1.97	
	Delta WM	Female	17	-0.035	0.255	-0.17	0.10	-0.40	0.52	
		Male	14	-0.131	0.275	-0.29	0.03	-0.67	0.31	
		Total	31	-0.078	0.264	-0.18	0.02	-0.67	0.52	0.110
	RT	Female	17	1.399	0.261	1.27	1.53	0.85	2.13	
		Male	14	1.398	0.232	1.26	1.53	1.05	1.93	
		Total	31	1.399	0.244	1.31	1.49	0.85	2.13	
	Delta RT	Female	17	-0.061	0.286	-0.21	0.09	-0.72	0.28	
		Male	14	-0.046	0.191	-0.16	0.06	-0.46	0.29	
		Total	31	-0.055	0.244	-0.14	0.04	-0.72	0.29	0.223
	RTSD	Female	17	0.528	0.128	0.46	0.59	0.29	0.81	
		Male	14	0.510	0.092	0.46	0.56	0.39	0.63	
		Total	31	0.520	0.112	0.48	0.56	0.29	0.81	

FA Rate, false alarm rate; A', sensitivity; B”, response Bias; WM, working memory; RT, Response Time; RTSD, Response Time Standard Deviation; SD, standard deviation; CI, confidence interval; Min, minimum; Max, maximum.

**Table 4:** Descriptive statistics and 95% CIs for cognitive-behavioral parameters in the auditory-verbal modality, in different time-blocks. The delta values are calculated as the second half of each block minus the first half of that block. The *P* values are computed by comparing the mean delta values with zero, using the one-sample t-test. A significantly positive mean delta value indicates an increase in the parameter over the 8-minute time of the block.

Time-block	Parameter	Sex	N	Mean	SD	95% CI		Min	Max	*P*
1	Hit Rate	Female	17	0.820	0.141	0.75	0.89	0.37	0.97	
		Male	14	0.848	0.135	0.77	0.93	0.53	1.00	
		Total	31	0.833	0.137	0.78	0.88	0.37	1.00	
	Delta Hit Rate	Female	17	-0.008	0.183	-0.10	0.09	-0.28	0.40	
		Male	14	-0.005	0.122	-0.08	0.07	-0.19	0.26	
		Total	31	-0.007	0.156	-0.06	0.05	-0.28	0.40	0.817
	FA Rate	Female	17	0.150	0.093	0.10	0.20	0.03	0.40	
		Male	14	0.098	0.067	0.06	0.14	0.02	0.28	
		Total	31	0.126	0.085	0.10	0.16	0.02	0.40	
	Delta FA Rate	Female	17	0.023	0.058	-0.01	0.05	-0.11	0.11	
		Male	14	0.024	0.071	-0.02	0.06	-0.07	0.15	
		Total	31	0.023	0.063	0.00	0.05	-0.11	0.15	0.047
	A'	Female	17	0.903	0.045	0.88	0.93	0.80	0.97	
		Male	14	0.930	0.039	0.91	0.95	0.85	0.98	
		Total	31	0.915	0.044	0.90	0.93	0.80	0.98	
	Delta A'	Female	17	-0.015	0.063	-0.05	0.02	-0.11	0.11	
		Male	14	-0.007	0.050	-0.04	0.02	-0.08	0.10	
		Total	31	-0.011	0.057	-0.03	0.01	-0.11	0.11	0.272
	B''	Female	17	0.012	0.430	-0.21	0.23	-0.70	0.70	
		Male	14	0.003	0.621	-0.36	0.36	-1.00	0.84	
		Total	31	0.008	0.515	-0.18	0.20	-1.00	0.84	
	WM	Female	17	1.341	0.274	1.20	1.48	0.65	1.78	
		Male	14	1.500	0.256	1.35	1.65	0.96	1.84	
		Total	31	1.413	0.274	1.31	1.51	0.65	1.84	
	Delta WM	Female	17	-0.062	0.385	-0.26	0.14	-0.66	0.80	
		Male	14	-0.057	0.313	-0.24	0.12	-0.54	0.59	
		Total	31	-0.060	0.349	-0.19	0.07	-0.66	0.80	0.346
	RT	Female	17	1.586	0.210	1.48	1.69	1.21	1.91	
		Male	14	1.667	0.187	1.56	1.78	1.38	2.02	
		Total	31	1.623	0.201	1.55	1.70	1.21	2.02	
	Delta RT	Female	17	-0.134	0.197	-0.23	-0.03	-0.56	0.15	
		Male	14	-0.050	0.252	-0.20	0.10	-0.60	0.26	
		Total	31	-0.096	0.224	-0.18	-0.01	-0.60	0.26	0.024
	RTSD	Female	17	0.467	0.129	0.40	0.53	0.23	0.70	
		Male	14	0.492	0.087	0.44	0.54	0.31	0.68	
		Total	31	0.478	0.111	0.44	0.52	0.23	0.70	

2	Hit Rate	Female	17	0.835	0.108	0.78	0.89	0.60	0.97	
		Male	14	0.900	0.090	0.85	0.95	0.67	1.00	
		Total	31	0.865	0.104	0.83	0.90	0.60	1.00	
	Delta Hit Rate	Female	17	0.028	0.130	-0.04	0.09	-0.27	0.22	
		Male	14	-0.032	0.127	-0.10	0.04	-0.25	0.28	
		Total	31	0.001	0.130	-0.05	0.05	-0.27	0.28	0.969
	FA Rate	Female	17	0.121	0.088	0.08	0.17	0.03	0.34	
		Male	14	0.100	0.050	0.07	0.13	0.04	0.23	
		Total	31	0.111	0.073	0.08	0.14	0.03	0.34	
	Delta FA Rate	Female	17	0.025	0.049	0.00	0.05	-0.06	0.13	
		Male	14	0.035	0.034	0.02	0.05	-0.02	0.08	
		Total	31	0.029	0.043	0.01	0.04	-0.06	0.13	0.001
	A'	Female	17	0.915	0.054	0.89	0.94	0.75	0.98	
		Male	14	0.944	0.032	0.93	0.96	0.88	0.98	
		Total	31	0.928	0.047	0.91	0.95	0.75	0.98	
	Delta A'	Female	17	0.002	0.045	-0.02	0.03	-0.11	0.07	
		Male	14	-0.023	0.046	-0.05	0.00	-0.13	0.06	
		Total	31	-0.009	0.047	-0.03	0.01	-0.13	0.07	0.298
	B''	Female	17	0.104	0.393	-0.10	0.31	-0.58	0.70	
		Male	14	-0.134	0.542	-0.45	0.18	-1.00	0.55	
		Total	31	-0.004	0.473	-0.18	0.17	-1.00	0.70	
	WM	Female	17	1.429	0.288	1.28	1.58	0.66	1.88	
		Male	14	1.600	0.201	1.48	1.72	1.19	1.81	
		Total	31	1.506	0.263	1.41	1.60	0.66	1.88	
	Delta WM	Female	17	0.006	0.277	-0.14	0.15	-0.66	0.45	
		Male	14	-0.132	0.276	-0.29	0.03	-0.67	0.44	
		Total	31	-0.056	0.281	-0.16	0.05	-0.67	0.45	0.272
	RT	Female	17	1.557	0.205	1.45	1.66	1.28	2.03	
		Male	14	1.649	0.221	1.52	1.78	1.31	2.04	
		Total	31	1.598	0.214	1.52	1.68	1.28	2.04	
	Delta RT	Female	17	0.012	0.198	-0.09	0.11	-0.32	0.36	
		Male	14	0.015	0.147	-0.07	0.10	-0.24	0.22	
		Total	31	0.013	0.174	-0.05	0.08	-0.32	0.36	0.681
	RTSD	Female	17	0.484	0.128	0.42	0.55	0.24	0.70	
		Male	14	0.479	0.083	0.43	0.53	0.36	0.65	
		Total	31	0.482	0.108	0.44	0.52	0.24	0.70	

3	Hit Rate	Female	17	0.887	0.107	0.83	0.94	0.63	1.00	
		Male	14	0.915	0.085	0.87	0.96	0.73	1.00	
		Total	31	0.900	0.097	0.86	0.94	0.63	1.00	
	Delta Hit Rate	Female	17	-0.066	0.078	-0.11	-0.03	-0.19	0.08	
		Male	14	-0.019	0.086	-0.07	0.03	-0.21	0.14	
		Total	31	-0.045	0.084	-0.08	-0.01	-0.21	0.14	0.006
	FA Rate	Female	17	0.126	0.109	0.07	0.18	0.03	0.49	
		Male	14	0.096	0.055	0.06	0.13	0.02	0.23	
		Total	31	0.113	0.089	0.08	0.15	0.02	0.49	
	Delta FA Rate	Female	17	-0.009	0.055	-0.04	0.02	-0.09	0.11	
		Male	14	0.009	0.043	-0.02	0.03	-0.07	0.06	
		Total	31	-0.001	0.050	-0.02	0.02	-0.09	0.11	0.911
	A'	Female	17	0.929	0.062	0.90	0.96	0.73	0.99	
		Male	14	0.950	0.032	0.93	0.97	0.86	1.00	
		Total	31	0.938	0.051	0.92	0.96	0.73	1.00	
	Delta A'	Female	17	-0.022	0.045	-0.05	0.00	-0.14	0.04	
		Male	14	-0.008	0.030	-0.03	0.01	-0.08	0.03	
		Total	31	-0.016	0.039	-0.03	0.00	-0.14	0.04	0.031
	B''	Female	17	-0.182	0.535	-0.46	0.09	-1.00	0.65	
		Male	14	-0.256	0.550	-0.57	0.06	-1.00	0.71	
		Total	31	-0.215	0.534	-0.41	-0.02	-1.00	0.71	
	WM	Female	17	1.521	0.338	1.35	1.69	0.56	1.91	
		Male	14	1.638	0.207	1.52	1.76	1.15	1.97	
		Total	31	1.574	0.288	1.47	1.68	0.56	1.97	
	Delta WM	Female	17	-0.115	0.233	-0.23	0.00	-0.50	0.23	
		Male	14	-0.055	0.193	-0.17	0.06	-0.53	0.17	
		Total	31	-0.088	0.214	-0.17	-0.01	-0.53	0.23	0.030
	RT	Female	17	1.534	0.209	1.43	1.64	1.12	1.91	
		Male	14	1.559	0.183	1.45	1.66	1.32	2.00	
		Total	31	1.545	0.195	1.47	1.62	1.12	2.00	
	Delta RT	Female	17	-0.039	0.168	-0.13	0.05	-0.42	0.20	
		Male	14	-0.001	0.136	-0.08	0.08	-0.23	0.27	
		Total	31	-0.022	0.153	-0.08	0.03	-0.42	0.27	0.432
	RTSD	Female	17	0.511	0.124	0.45	0.57	0.30	0.69	
		Male	14	0.458	0.124	0.39	0.53	0.19	0.60	
		Total	31	0.487	0.125	0.44	0.53	0.19	0.69	

4	Hit Rate	Female	17	0.893	0.086	0.85	0.94	0.63	1.00	
		Male	14	0.913	0.104	0.85	0.97	0.65	1.00	
		Total	31	0.902	0.094	0.87	0.94	0.63	1.00	
	Delta Hit Rate	Female	17	-0.001	0.112	-0.06	0.06	-0.19	0.20	
		Male	14	-0.089	0.108	-0.15	-0.03	-0.27	0.14	
		Total	31	-0.041	0.117	-0.08	0.00	-0.27	0.20	0.063
	FA Rate	Female	17	0.145	0.141	0.07	0.22	0.04	0.64	
		Male	14	0.074	0.036	0.05	0.09	0.02	0.16	
		Total	31	0.113	0.112	0.07	0.15	0.02	0.64	
		Female	17	0.023	0.058	-0.01	0.05	-0.05	0.14	
		Male	14	0.018	0.047	-0.01	0.04	-0.09	0.08	
		Total	31	0.021	0.052	0.00	0.04	-0.09	0.14	0.033
	A'	Female	17	0.927	0.054	0.90	0.95	0.76	0.98	
		Male	14	0.957	0.029	0.94	0.97	0.89	1.00	
		Total	31	0.940	0.046	0.92	0.96	0.76	1.00	
	Delta A'	Female	17	-0.005	0.041	-0.03	0.02	-0.09	0.05	
		Male	14	-0.030	0.039	-0.05	-0.01	-0.09	0.07	
		Total	31	-0.017	0.041	-0.03	0.00	-0.09	0.07	0.033
	B''	Female	17	-0.106	0.412	-0.32	0.11	-1.00	0.40	
		Male	14	-0.205	0.611	-0.56	0.15	-1.00	0.64	
		Total	31	-0.151	0.505	-0.34	0.03	-1.00	0.64	
	WM	Female	17	1.495	0.316	1.33	1.66	0.53	1.81	
		Male	14	1.680	0.205	1.56	1.80	1.19	1.97	
		Total	31	1.578	0.283	1.47	1.68	0.53	1.97	
	Delta WM	Female	17	-0.049	0.253	-0.18	0.08	-0.55	0.34	
		Male	14	-0.214	0.253	-0.36	-0.07	-0.63	0.45	
		Total	31	-0.123	0.263	-0.22	-0.03	-0.63	0.45	0.014
	RT	Female	17	1.513	0.249	1.38	1.64	1.09	1.92	
		Male	14	1.520	0.206	1.40	1.64	1.19	1.83	
		Total	31	1.516	0.227	1.43	1.60	1.09	1.92	
	Delta RT	Female	17	-0.010	0.167	-0.10	0.08	-0.22	0.28	
		Male	14	-0.047	0.204	-0.16	0.07	-0.52	0.31	
		Total	31	-0.026	0.182	-0.09	0.04	-0.52	0.31	0.425
	RTSD	Female	17	0.456	0.119	0.39	0.52	0.25	0.66	
		Male	14	0.440	0.107	0.38	0.50	0.33	0.74	
		Total	31	0.449	0.112	0.41	0.49	0.25	0.74	

5	Hit Rate	Female	17	0.875	0.094	0.83	0.92	0.70	0.97	
		Male	14	0.915	0.100	0.86	0.97	0.67	1.00	
		Total	31	0.893	0.097	0.86	0.93	0.67	1.00	
	Delta Hit Rate	Female	17	-0.043	0.150	-0.12	0.03	-0.30	0.19	
		Male	14	-0.002	0.122	-0.07	0.07	-0.35	0.17	
		Total	31	-0.025	0.138	-0.08	0.03	-0.35	0.19	0.323
	FA Rate	Female	17	0.131	0.122	0.07	0.19	0.04	0.57	
		Male	14	0.077	0.043	0.05	0.10	0.00	0.16	
		Total	31	0.106	0.097	0.07	0.14	0.00	0.57	
	Delta FA Rate	Female	17	0.022	0.062	-0.01	0.05	-0.10	0.10	
		Male	14	0.019	0.045	-0.01	0.05	-0.04	0.10	
		Total	31	0.021	0.054	0.00	0.04	-0.10	0.10	0.041
	A'	Female	17	0.924	0.061	0.89	0.96	0.71	0.98	
		Male	14	0.955	0.035	0.93	0.98	0.88	0.99	
		Total	31	0.938	0.053	0.92	0.96	0.71	0.99	
	Delta A'	Female	17	-0.019	0.062	-0.05	0.01	-0.12	0.09	
		Male	14	-0.006	0.043	-0.03	0.02	-0.13	0.06	
		Total	31	-0.013	0.054	-0.03	0.01	-0.13	0.09	0.189
	B''	Female	17	-0.051	0.443	-0.28	0.18	-0.69	0.67	
		Male	14	-0.162	0.614	-0.52	0.19	-1.00	1.00	
		Total	31	-0.101	0.520	-0.29	0.09	-1.00	1.00	
	WM	Female	17	1.487	0.313	1.33	1.65	0.47	1.81	
		Male	14	1.676	0.236	1.54	1.81	1.18	1.93	
		Total	31	1.572	0.292	1.47	1.68	0.47	1.93	
	Delta WM	Female	17	-0.130	0.371	-0.32	0.06	-0.68	0.47	
		Male	14	-0.044	0.277	-0.20	0.12	-0.82	0.32	
		Total	31	-0.091	0.330	-0.21	0.03	-0.82	0.47	0.134
	RT	Female	17	1.475	0.245	1.35	1.60	1.04	1.90	
		Male	14	1.497	0.174	1.40	1.60	1.16	1.81	
		Total	31	1.485	0.213	1.41	1.56	1.04	1.90	
	Delta RT	Female	17	-0.039	0.172	-0.13	0.05	-0.49	0.19	
		Male	14	-0.094	0.163	-0.19	0.00	-0.30	0.23	
		Total	31	-0.064	0.168	-0.13	0.00	-0.49	0.23	0.043
	RTSD	Female	17	0.422	0.128	0.36	0.49	0.24	0.70	
		Male	14	0.449	0.067	0.41	0.49	0.29	0.55	
		Total	31	0.434	0.104	0.40	0.47	0.24	0.70	

FA Rate, false alarm rate; A', sensitivity; B”, response Bias; WM, working memory; RT, Response Time; RTSD, Response Time Standard Deviation; SD, standard deviation; CI, confidence interval; Min, minimum; Max, maximum.

**Table 5:** Pearson correlations (*R*) between response times and four cognitive measures in different intervention groups (*n* of each coefficient = 31).

Modality	Intervention		Hit Rate	FA Rate	A'	WM
Visuospatial	Silence	*R*	-0.597	0.346	-0.568	-0.586
		*P*	<0.0005	0.056	0.001	0.001
	Pure tone	*R*	-0.470	0.230	-0.369	-0.439
		*P*	0.008	0.214	0.041	0.013
	BB 10 Hz	*R*	-0.274	0.284	-0.310	-0.327
		*P*	0.136	0.122	0.089	0.072
	BB 16 Hz	*R*	-0.488	0.350	-0.548	-0.551
		*P*	0.005	0.054	0.001	0.001
	BB 40 Hz	*R*	-0.475	0.451	-0.527	-0.525
		*P*	0.007	0.011	0.002	0.002

Auditory-Verbal	Silence	*R*	-0.423	0.047	-0.290	-0.344
		*P*	0.018	0.803	0.114	0.058
	Pure tone	*R*	-0.244	-0.107	-0.049	-0.083
		*P*	0.185	0.566	0.795	0.657
	BB 10 Hz	*R*	-0.410	-0.248	-0.110	-0.192
		*P*	0.022	0.179	0.554	0.301
	BB 16 Hz	*R*	-0.159	-0.078	-0.042	-0.071
		*P*	0.392	0.675	0.821	0.705
	BB 40 Hz	*R*	-0.445	0.179	-0.425	-0.424
		*P*	0.012	0.334	0.017	0.017

FA Rate, false alarm rate; A', sensitivity; WM, working memory.

**Table 6:** Pearson correlations (*R*) between response times and four cognitive measures in various time-blocks (n for each coefficient = 31).

Modality	Time		Hit Rate	FA Rate	A'	WM
Visuospatial	1	*R*	-0.392	0.309	-0.440	-0.446
		*P*	0.029	0.091	0.013	0.012
	2	*R*	-0.530	0.389	-0.533	-0.548
		*P*	0.002	0.030	0.002	0.001
	3	*R*	-0.472	0.366	-0.529	-0.510
		*P*	0.007	0.043	0.002	0.003
	4	*R*	-0.464	0.268	-0.422	-0.475
		*P*	0.009	0.145	0.018	0.007
	5	*R*	-0.400	0.210	-0.344	-0.382
		*P*	0.026	0.258	0.058	0.034

Auditory-Verbal	1	*R*	-0.355	-0.094	-0.288	-0.297
		*P*	0.050	0.616	0.117	0.104
	2	*R*	-0.262	-0.153	-0.082	-0.122
		*P*	0.155	0.412	0.663	0.514
	3	*R*	-0.323	-0.045	-0.145	-0.191
		*P*	0.076	0.809	0.435	0.305
	4	*R*	-0.258	-0.025	-0.129	-0.150
		*P*	0.161	0.892	0.488	0.419
	5	*R*	-0.340	-0.116	-0.089	-0.149
		*P*	0.061	0.533	0.635	0.423

FA Rate, false alarm rate; A', sensitivity; WM, working memory.

## Data Availability

The data are available from Dr. Vahid Rakhshan upon reasonable request.
